RETRACTED

# Deceptology in cancer and vaccine sciences: Seeds of immune destruction‐mini electric shocks in mitochondria: Neuroplasticity‐electrobiology of response profiles and increased induced diseases in four generations – A hypothesis

**DOI:** 10.1002/ctm2.215

**Published:** 2020-12-19

**Authors:** Mahin Khatami

**Affiliations:** ^1^ Inflammation, Aging and Cancer, National Cancer Institute (NCI) the National Institutes of Health (NIH) (Retired) Bethesda Maryland USA

**Keywords:** adjuvant, aluminum, antigen overload, autism, autoimmune disease, cancer bioenergetics, constituent and inducible receptors, deceptology, fetus tissue, Gates vaccines, gene‐environment‐immune, genomics, glyphosate, histidine‐histamine, HPV, hypoxia, immune‐privileged, immune‐responsive, inflammation, intellectual harassment, mercury, mini electrical shocks, mitochondria, molecular sink holes, neurodegenerative diseases, pathogen‐specific vaccines, philanthropists, placenta, policy makers, Rockefeller medicine, therapy, trophoblast, tumoricidal, tumorigenic, vaccine incipient, Yin and Yang of immunity

## Abstract

From Rockefeller's support of patent medicine to Gates' patent vaccines, medical establishment invested a great deal in intellectual ignorance. Through the control over medical education and research it has created a public illusion to prop up corporate profit and encouraged the lust for money and power. An overview of data on cancer and vaccine sciences, the status of Americans' health, a survey of repeated failed projects, economic toxicity, and heavy drug consumption or addiction among young and old provide compelling evidence that in the twentieth century nearly all classic disease categories (congenital, inheritance, neonatal, or induced) shifted to increase induced diseases. Examples of this deceptology in ignoring or minimizing, and mocking fundamental discoveries and theories in cancer and vaccine sciences are attacks on research showing that (a), effective immunity is responsible for defending and killing pathogens and defective cancerous cells, correcting and repairing genetic mutations; (b) viruses cause cancer; and (c), abnormal gene mutations are often the consequences of (and secondary to) disturbances in effective immunity. The outcomes of cancer reductionist approaches to therapies reveal failure rates of 90% (+/‐5) for solid tumors; loss of over 50 million lives and waste of $30‐50 trillions on too many worthless, out‐of‐focus, and irresponsible projects. Current emphasis on vaccination of public with pathogen‐specific vaccines and ingredients seems new terms for drugging young and old. Cumulative exposures to low level carcinogens and environmental hazards or high energy electronic devices (EMF; 5G) are additional triggers to vaccine toxicities (antigen‐mitochondrial overload) or “seeds of immune destruction” that create mini electrical shocks (molecular sinks holes) in highly synchronized and regulated immune network that retard time‐energy‐dependent biorhythms in organs resulting in causes, exacerbations or consequences of mild, moderate or severe immune disorders. Four generations of drug‐dependent Americans strongly suggest that medical establishment has practiced decades of intellectual deception through its claims on “war on cancer”; that cancer is 100, 200, or 1000 diseases; identification of “individual” genetic mutations to cure diseases; “vaccines are safe”. Such immoral and unethical practices, along with intellectual harassment and bullying, censoring or silencing of independent and competent professionals (“Intellectual Me Too”) present grave concerns, far greater compared with the sexual harassment of ‘Me Too’ movement that was recently spearheaded by NIH. The principal driving forces behind conducting deceptive and illogical medical/cancer and vaccine projects seem to be; (a) huge return of investment and corporate profit for selling drugs and vaccines; (b) maintenance of abusive power over public health; (c) global control of population growth via increased induction of diseases, infertility, decline in life‐span, and death.

RETRACTED

An overview of accidental discoveries that we established and extended since 1980s, on models of acute and chronic ocular inflammatory diseases, provides series of the first evidence for a direct link between inflammation and multistep immune dysfunction in tumorigenesis and angiogenesis. Results are relevant to demonstrate that current emphasis on vaccinating the unborn, newborn, or infant would induce immediate or long‐term immune disorders (eg, low birth weight, preterm birth, fatigue, autism, epilepsy/seizures, BBB leakage, autoimmune, neurodegenerative or digestive diseases, obesity, diabetes, cardiovascular problems, or cancers). Vaccination of the unborn is likely to disturb trophoblast‐embryo‐fetus‐placenta biology and orderly growth of embryo‐fetus, alter epithelial‐mesenchymal transition or constituent‐inducible receptors, damage mitochondria, and diverse function of histamine‐histidine pathways. Significant increased in childhood illnesses are likely due to toxicities of vaccine and incipient (eg, metals [Al, Hg], detergents, fetal tissue, DNA/RNA) that retard bioenergetics of mitochondria, alter polarization‐depolarization balance of tumoricidal (Yin) and tumorigenic (Yang) properties of immunity.

Captivated by complex electobiology of immunity, this multidisciplinary perspective is an attempt to initiate identifying bases for increased induction of immune disorders in three to four generations in America. We hypothesize that (a) gene‐environment‐immune biorhythms parallel neuronal function (brain neuroplasticity) with super‐packages of inducible (adaptive or horizontal) electronic signals and (b) autonomic sympathetic and parasympathetic circuitry that shape immunity (Yin‐Yang) cannot be explained by limited genomics (innate, perpendicular) that conventionally explain certain inherited diseases (eg, sickle cell anemia, progeria). Future studies should focus on deep learning of complex electrobiology of immunity that requires differential bioenergetics from mitochondria and cytoplasm. Approaches to limit or control excessive activation of gene‐environment‐immunity are keys to assess accurate disease risk formulations, prevent inducible diseases, and develop universal safe vaccines that promote health, the most basic human right.

RETRACTED

## Graphical abstract

Schematic representation of cause, exacerbation and consequence of vaccines‐induced diverse immune disorders in immune‐responsive or immune‐privileged tissues. It depicts that vaccination of the unborn, alter biology of trophoblast‐embryo‐fetus‐placenta and orderly growth and development affecting epithelial‐mesenchymal transition, proper expression of constituent‐inducible receptor molecules; consequently influence immunity of newborn, infant, children and adults. Vaccine‐induced impaired organ development and immunity include impaired mitochondrial function (mitophagy), tissue bioenergetics, loss of balance in Yin (tumoricidal) and Yang (tumorigenic) pathways and altered metabolic‐neuronal‐hormonal activities as bases for increased induced diseases in young and old.

Hypothesis: (a) gene‐environment‐induced immune responses (adaptive, horizontal, immune neuroplasticity) parallel neuronal function; (b) complex autonomic sympathetic‐parasympathetic and electrobiology of effective immunity (or immune disorders) cannot be explained by limited genomics (innate, perpendicular) that are known to explain certain inherited disease.

**Abbreviations**
ACIP: Advisory Committee on Immunization Practices
ALS: amyotrophic lateral sclerosis
ASD: autism spectrum disorders
CALTs: conjunctival associated lymphoid tissues
CICP: countermeasures Injury Compensation Program
CTAB: cetyl‐trimethyl‐ammonium bromide
FGF: fibroblast growth factor
FLOA: fluorescinated ovalbumin
ILs: interleukins
IRAK: interleukin receptor‐associated kinase
MMPs: membrane metalloproteases
mTOR: mammalian target of rapamycin
PHT1: peptide‐histidine transporter 1
PTH: parathyroid hormone
SIDS: sudden infant death syndrome
SODs: superoxide dismutases
STAT: signal transduction and activation of transcription
TNFRs: tumor necrosis factor receptors
VAERS: Vaccine Adverse Event Reporting System
VRBPAC: Vaccines and Related Biological Products Advisory Committee

RETRACTED

## 1 INTRODUCTION

*A great deal of intelligence can be invested in ignorance when the need for illusion is deep!* Saul Bellow

*We have remained in the dark long enough to talk about the light*. Sohrab Sepehri

In the 20th century, the patent medical establishment, led by a coalition of Governments‐Big Pharma and Venture‐Capitalists‐‘Philanthropists’ (disease investors) invested a great deal on intellectual ignorance in medical education and research projects because the need for a public illusion that would generate corporate profit seemed deep and dark. The illusion fed on medical projects initiated by the twisted and profitable cholesterol story and extended to other fabricated and expensive projects on cancer and vaccine sciences that repeatedly failed. Significant increased in the sick population in America (young and old), heavy consumption and addiction to drugs and the current emphasis to vaccinate the public with pathogen‐specific vaccines demonstrate that motives of the medical establishment in conducting too many intellectually fraudulent projects are diametrically opposing the mission to improve public health by preventing diseases or saving lives [reviewed in refs. ^1^, ^2^, ^3^, ^4^, ^5^, ^6^, ^7^, ^8^, ^9^, ^10^, ^11^, ^12^, ^13^, ^14^, ^15^, ^16^, ^17^, ^18^, ^19^, ^20^, ^21^, ^22^, ^23^, ^24^, ^25^].

To better appreciate the extent of this intellectual deception, fraud, and chaos in conducting scientific/clinical projects that were practiced by the medical establishment against public health, the author chose the word of ”deceptology.” Deceptology in medical/cancer and vaccine sciences refers to a combination of adjectives such as deception, prank, magic, scam, fraud, cons, and propaganda; fear‐mongering, bias, nepotism, and heavy bribes in conducting projects. Tremendous financial gain and absolute power to control public health were accomplished by endless intellectual deception (scientific/medical Ponzi schemes) in marketing failed projects. As detailed below, novel ideas and discoveries are routinely hijacked, fragmented, and used as a front to collect funding from taxpayers. Decisions on expensive and out‐of‐focus projects are associated with ignoring medical morals or ethics and conflict of interest, while practicing heavy intellectual bullying, harassing, and silencing of independent and competent professionals^1^, ^2^, ^3^, ^4^, ^5^, ^6^, ^7^, ^8^, ^9^, ^10^, ^11^, ^12^.

RETRACTED

The “medical establishment” refers to a highly organized and powerful group, a hierarchy with military‐like structure that functions like an elite tribe and operates globally. The medical establishment is an intimate and co‐dependent partnership between decision makers in governments (eg, NIH‐FDA‐CDC‐DHHS, WHO)*, Big Pharma, venture capitalists ‘philanthropists’ (disease investors), medical/cancer research and treatment centers, organizations (eg, AMA, AACR, ASCO, ACS, APS), insurance companies, major food industry players and the main stream media outlets that collectively control the marketing of foods, drugs, and vaccines. Globally, the estimated total number of members in medical establishment including the world's largest lobbying and support groups, handlers/cronies (institutes’ directors, department chairs, and staff) is 4–6 millions. In this power structure, the role of policymakers, with/without scientific/medical backgrounds who are largely influenced (including monetarily) by lobbying groups cannot be ignored. This power structure channels funds and sponsors legislations on behalf of the medical establishment (eg, recent actions to mandate vaccination “*Give Kids a Shot*”; ‘Moonshot’ initiative [2016] that increased funding for NCI/NIH by $1.6 B for HPV vaccines and cancer research; or Cancer Act by President Nixon [1970] that increased funding for cancer research by 1.6 B to resolve cancer problem in 8 years!!).^1^, ^7^, ^8^, ^12^, ^18^ †’‡

Details on financial structures and cycles of collaborations between governmental agencies, pharmaceutical companies, and medical education programs on the promotion of drugs are provided in an informative book by Marcia Angell, MD (past Editor‐In‐Chief of *New England Journal of Medicine*).^2^ It describes how drug companies operate within this system [“*Buying Influence‐How the Industry Makes Sure It Gets Its Way…Bribing Doctors—or Nurturing Consultants…*”] by selling drugs that scientists/physicians advocate on behalf of industry; and by charging taxpayers twice, once for supporting research of government‐academia and again paying for prescription drugs at prices that are set by manufacturers. In another instructive book, John Geyman, MD^3^ describes the market‐driven healthcare that changed medical practices; that physicians frequently ignore the principles of the medical profession (patient welfare, patient autonomy, social justice, medical ethics, and moral values of healthcare) and doing no harm. Geyman demonstrates that physicians routinely misdiagnose or over‐diagnose diseases and prescribe drugs that are promoted by Big Pharma, while downplaying conflicts of interest and ignoring medical ethics by accepting fees for consultations and honoraria to lecture on behalf of drug companies who are also organizers of continuing medical education programs.^3^ In a series of informative books, Harris Coulter, MD, describes the history and philosophical approaches to medicine from the time of Hippocrates to the 20th century and the conflicts between the two systems of empiricism and rationalism,^15^, ^16^ or as we have described the differences between integrated and reductionist approaches to the medical sciences.^1^, ^5^, ^8^, ^10^, ^11^, ^12^, ^20^ In another comprehensive publication, by an independent vaccine and health journalist, Jeremy Hammond describes the FDA vaccine approval process “*The Government Is the Vaccine Industry*”. Hammond details how the perception that the government is serving on behalf of the public is far from the truth.^4^ Suzanne Humphries, MD and Roman Bystriany^17^ in an eye‐opening book describe the history behind polio vaccines and induction of diseases despite protests against vaccination since 1919. The quotation by Eustace Mullins that public vaccination is “*Murder* by Injection” (reviewed in ref. 17) has scientific merits as we describe below the toxicity of current drugs and vaccines. In another report,^18^ Brandon Turbeville describes that The American Legislative Exchange Council (ALEC), a “non‐profitable organization” is a “*driving force behind the current drive for mandatory vaccine bills … a source of enormous profits for drug manufacturers*…”. Details on operation of ALEC, along with names of companies, contributors, beneficiaries within and outside government, and the agenda for vaccine mandates are provided in this report.^18^

RETRACTED

This multidimensional perspective/hypothesis is a brief overview of identifying a century of intellectual deception, chaos, and fraud that the medical establishment practiced in conducting failed cancer and vaccine sciences. Ignoring the truth about the motives behind too many ill‐conceived, reckless, and failed projects that led to the loss of millions of precious lives and creation of three to four generations of sick and drug‐dependent people and the huge economic burden to the society are no longer tolerable, acceptable, or sustainable. The first steps to switching the disease‐care mentality of the medical establishment are to present sufficient biological evidence to reveal the the hidden agenda behind this massive intellectual deception in conducting medical/cancer and vaccine sciences. The hidden agenda seeks to deny health to the public by chipping away and destroying the body's natural immunity in an effort to regulate population growth, maintain an ill, easily controlled worker population, and effectuate wealth transfer from the public to the establishment. Future scientific directions should include cleaning up the massive misinformation (scientific noise and frauds) on cancer and vaccine sciences, while focusing on designs of cost‐effective systematic and logical studies to promote immunity, assess accurate risk formulations, develop safe/universal vaccines with the goal to improve health and prevent diseases for a healthier and more productive society.

RETRACTED

## 2 FROM ROCKEFELLER MEDICINE TO GATES VACCINES: REDUCTIONIST AND FRAUD APPROACHES TO CANCER AND VACCINE SCIENCES. INDUCTION OF DISEASES IN YOUNG AND OLD FOR DRUG SALE

In 1900s, the Rockefeller and other “philanthropists” (who should be identified as “disease investors”) supported medical school education programs with an eye toward influencing drug development and sale. The major drug business initiated with an intellectually twisted story on cholesterol‐lowering drugs that continue to generate billions of dollars for the industry. The side‐effects of such drugs made millions of older individuals sick and brought additional profits for drug manufacturers and food industry.^1^, ^6^, ^7^, ^8^ § In a recent documentary, Aseem Malhotra, MD, noted it was “*time for a full public parliamentary inquiry into the controversial drug and to fully expose the great cholesterol and statin con*.”^6^ ** The ill‐designed studies that promoted and educated physicians for use of cholesterol inhibitors became bases for a shared Nobel prize by Brown and Goldstein and development of statins and their derivatives.^6^ ††

A century ago, the leading causes of death were pneumonia/influenza, tuberculosis, and diarrhea followed by heart disease and stroke. In all likelihood, at the turn of past century, heart disease and stroke were also the consequences of serious infections that shortened life expectancy, particularly in poor neighborhoods, and in the absence of antibiotics and better hygiene. Available statistics show that in 1900s, cancer occurred occasionally, as a genetic disorder (inherited disease category) at the rate of 5%.^1^, ^5^, ^8^

Eight decades ago the National Institutes of Health (NIH) or “the hidden crown jewel of corruption in the government”^8^ were established and received funding from taxpayers; and in collaborations with other governmental health agencies and centers within DHHS, had the “mission” to improve public health, prevent and treat diseases, and save lives.^1^, ^8^, ^12^, ^13^ However, despite improved hygiene and development of antibiotics and modern diagnostic technologies, the health status of Americans became significantly lower compared with the previous two to four generations at the same age and lowest compared with other developed nations. Since 1955s, after public was introduced to virus‐contaminated polio vaccines, cancer incident and mortality and numerous other diseases sharply increased, particularly in America. In 2013, the American Association for Cancer Research (AACR, among the largest cancer organizations and lobbying group for establishment) announced that one‐third of women (33%) and half of men (50%) develop cancer in their life‐time.^1^, ^5^, ^8^, ^12^, ^13^, ^24^

Major associated factors in the increased induction of diseases, shorten life expectancy or death in America are combinations of consumption of too many drugs, reductionist approaches to cancer research and therapy, as well as toxicities of vaccines that target the unborn, newborn, infant, or individuals (young and old) who are immune‐compromised (see below). Decision makers in medicine, major food and drug industry, or agricultural and electronic companies constantly design, advertise, and encourage public to use and be exposed to low level carcinogens (eg, glyphosate/ herbicides, pesticides, food additives and preservatives, artificial sweeteners, GMOs, chemical, biological and environmental hazards, or high energy electronic gadgets [4/5G devices]) that cumulatively weaken and interfere with the amazing electrobiology/ biorhythms that shape immunity and causing induction of mild, moderate or severe immune disorders.^1^, ^5^, ^6^, ^7^, ^8^, ^9^, ^10^, ^12^, ^13^, ^17^, ^18^, ^19^, ^20^, ^21^, ^22^, ^23^, ^24^, ^25^, ^26^, ^27^, ^28^, ^29^, ^30^, ^31^, ^32^, ^33^, ^34^, ^35^, ^36^, ^37^, ^38^, ^39^, ^40^, ^41^, ^42^, ^43^, ^44^, ^45^, ^46^, ^47^, ^48^, ^49^, ^50^ Objections, debates, questions, or suggested solutions on cancer or vaccine projects and clinical trials by independent and competent scientists are ignored or perceived as “dangerous” by decision makers^1^, ^2^, ^3^, ^4^, ^5^, ^6^, ^7^, ^8^, ^9^, ^10^, ^11^, ^12^, ^17^, ^22^ (Khatami, NCI/NIH scientific and legal documents, since 1998).

RETRACTED

In brief, the reductionist approach to cancer sciences is the real “dangerous” intellectual deception that made solving cancer a profitable myth‐making machine for the medical establishment.

Recently, we presented evidence that cancer is an induced disease of the 20th century, created by the medical establishment by allowing baby boomers to consume virus‐contaminated polio vaccines since 1955s.^1^, ^5^ We also presented evidence that, unlike popularized notions that cancer is 100, 200, or 1000 diseases, cancer is only one disease; the severely disrupted loss of highly regulated biorhythms of effective immunity, provided through tumoricidal (Yin) and tumorigenic (Yang) arms (autonomic sympathetic and parasympathetic) of acute inflammation.^5^

In this multidisciplinary perspective, we further provide evidence that nearly all clinically and pathologically established disease categories (neonatal, hereditary, congenital, and induced) that occasionally occurred at the rates of 1‐5% in the past century, have been shifted to increase the population of induced diseases in young and old. To achieve maximum disease status, particularly in America medical establishment employed combined methods of (a) heavy advertisements for the consumption of numerous drugs; (b) frequent vaccination of young and old with pathogen‐specific vaccines; and (c) cumulative exposures of public to environmental hazards.

Major methods that establishment continue to employ on utilizing reductionist approaches to cancer and vaccine projects that created tremendous misunderstanding, misinformation, debates, and controversies and resulted in increased diseases in young and old are listed below:^1^, ^2^, ^3^, ^4^, ^5^, ^6^, ^7^, ^8^, ^9^, ^10^, ^11^, ^12^, ^13^, ^14^, ^15^, ^16^, ^17^, ^18^, ^19^, ^20^, ^21^, ^22^, ^23^, ^24^, ^25^, ^26^, ^27^, ^28^, ^29^, ^30^, ^31^, ^32^, ^33^, ^34^, ^35^, ^36^, ^37^, ^38^, ^39^, ^40^, ^41^, ^42^, ^43^, ^44^, ^45^, ^46^, ^47^, ^48^, ^49^, ^50^, ^51^, ^52^, ^53^, ^54^, ^55^, ^56^, ^57^, ^58^, ^59^, ^60^, ^61^, ^62^, ^63^, ^64^, ^65^, ^66^, ^67^, ^68^, ^69^, ^70^, ^71^, ^72^, ^73^, ^74^, ^75^, ^76^, ^77^, ^78^, ^79^, ^80^, ^81^, ^82^, ^83^ §§’***’†††

- Definitions of inflammation/immunity, whether inflammation is protective in preventing cancer or it causes cancer;
- Identifying too many genetic mutations to develop and sell drugs (eg, monoclonal antibodies, inhibitors of growth factors);
- Claims of “targeted” therapy, “personalized” or “precision” medicine, or immunotherapy;
- Claims that “vaccines are safe,” with little serious safety and efficacy tests. Vaccine manufacturers have no liability or responsibility toward vaccine injuries;
- Incentives and royalties that scientists/physicians receive for advocating pathogen‐specific vaccines (eg, flu, HPV, meningitis, shingles, Hep a, b, c, MMR, EBOLA, ZIKA) or the “upcoming coronavirus vaccines”; as well as efforts to minimize voices of concern about vaccines safety;
- Heavy propaganda on the consumption of too many drugs for minor or major health conditions (eg, headache, muscle pain, allergies, depression, mood swings, cholesterol, indigestion, colitis, gastritis, sleep disorders, or cancers)

With regard to vaccines, Maurice Hilleman who developed several vaccines at Merck, in an interesting interview stated that “*vaccines have to be considered the bargain basement technology for the twentieth century*.”‡‡‡

One of the most dangerous plans of the establishment is the heavy propaganda campaign to vaccinate the unborn, newborn, infant, toddler, and teenagers with a total of 72 doses of 16 different pathogen‐specific vaccines by the time they are 18 years old.

RETRACTED

As detailed below, the presence of active or inactive specific pathogens and adjuvants in current vaccines are hypothesized as causes, aggregations‐exacerbations, and consequences of significant increased in immune disorders in young and old in the twentieth century,^1^, ^5^, ^8^, ^20^, ^40^, ^41^, ^42^, ^43^, ^44^, ^45^, ^46^, ^47^, ^48^, ^49^, ^50^, ^51^, ^52^, ^53^, ^54^, ^55^, ^56^, ^57^, ^58^, ^59^, ^60^, ^61^, ^62^, ^63^, ^64^, ^65^, ^66^, ^67^, ^68^, ^69^, ^70^, ^71^, ^72^, ^73^, ^74^, ^75^, ^76^, ^77^, ^78^, ^79^, ^80^, ^81^, ^82^, ^83^, ^84^, ^85^, ^86^, ^87^, ^88^, ^89^, ^90^ §§§ (Figure 1).

**FIGURE 1:** Schematic representation that current pathogen‐specific vaccines and incipient given to unborn (fetus), newborn or infant (age 0 to 24 mons), toddler or children (2‐16 years) are causes, exacerbations (aggregations) or consequences of development of a wide range of immune disorders that are often features of age‐associated chronic illnesses. Vaccination of unborn is depicted to lead to SIDS, preterm birth or low weight at birth, and associated underdeveloped immunity as bases for increased mortality and induction of childhood diseases. It depicts that current vaccines and metal‐containing ingredients are seeds of immune destruction, particularly affecting mitochondria and oxido‐redox potentials and immune‐metabolic‐hormonal‐neuronal activities. The scheme also represents that current vaccines and incipient shift/increase the classic categories of disease (inheritance, congenital, neonatal, and induced) to induced diseases. See text

## 3 IGNORING, WHILE ABUSING FUNDAMENTAL DISCOVERIES AND THEORIES OF IMMUNITY: CAUSES AND CONSEQUENCES OF DISEASES OR CANCER

*For evil to flourish, all that is needed is for good people to do nothing*. Edmund Burke.

The ability of inflammatory cells to destroy cancerous cells was first observed by Ilya Metchnikoff in the 19th century when the microscope was invented. Metchnikoff's report on phagocytic properties of inflammatory cells was the basis to study innate immunity. Paul Ehrlich also established the concept of antigen‐antibody complementarities and basis to study adaptive immunity. In 1908, the Nobel prize was shared between Ehrlich and Metchnikoff for their pioneering work in immunology and host defense mechanisms (reviewed in refs. ^1^, ^8^).

### 3.1 Initiators of cancer (tumor) growth and theory of immune surveillance

In 1910‐1911, the important and careful studies of Peyton Rous led to the discovery that viruses induce cancer. The main factor that was transmissible in chicken leukemia, lymphoma, sarcoma, and other neoplasms was a filterable virus (reviewed in refs. ^1^, ^8^, ^20^). Rous’ visionary work demonstrated the cumulative effects of the “initiators” in carcinogenesis. The integrated and generalized description of “initiators” in carcinogenesis that Rous defined was later extended and supported by the important theory of immune surveillance of Burnet in 1957^48^ and by our accidental discoveries (1980s) on direct evidence for cumulative effects of immune disruptors (antigens) in the initiation of multistep tumorigenesis and angiogenesis. Our earlier discoveries led to definitions of the Yin‐Yang‐like interplay of inflammation/immunity in the maintenance of health or induction and progression of nearly all acute and chronic diseases including site‐specific cancers (see below)^1^, ^5^, ^8^, ^20^, ^24^, ^25^, ^26^, ^41^, ^42^, ^43^, ^44^, ^45^, ^46^, ^47^, ^49^, ^50^, ^51^, ^52^ (Figure 2).

RETRACTED

**FIGURE 2:** Schematic representation that inflammation and aging are co‐risk factors in developmental phases of immune dysfunction in multistep tumorigenesis and angiogenesis. The left panel depicts initial stages of our ‘accidental’ discoveries on inflammation‐induced identifiable immune dysfunction in ocular tissue responses during (a) acute phase responses or self‐terminating inflammation (reversible); (b) intermediate phase, down‐regulation phenomenon accompanied with mild tissue atrophy and neovascularization (potentially reversible); and (c) chronic phase, induction of massive lymphoid hyperplasia and tumorigenesis and angiogenesis (irreversible?). The right panel represents chronic inflammation and continued stages of tissue growth (d,e), advancing to cancer malignancies and angiogenesis in site‐specific tissue. The complex scheme demonstrates that majorities of translational medicine and clinical trials are conducted in identification of endless damaged molecules at advanced stages of carcinogenesis for drug development and therapy (red arrows in phase e, ‘cancer tsunami’). Modified from Exp Opin Biol Ther; Informa Healthcare, 2011.^47^ All Rights reserved

The immune surveillance theory of Burnet was based on a decade of extensive analyses and integration of data from several scientific disciplines such as developmental biology, embryology, immunology, pathophysiology, and oncology of his era. Unlike the current reductionist approaches to cancer and vaccine sciences, Burnet realized that scientists like himself “*believe that at every stage in scientific development it is necessary to provide the best available generalizations as a guide to effective work, both in the application of knowledge to human needs and in the planning of future research….”*. Burnet explained that”*…Cancer is a negative condition‐ a manifestation of the breakdown in one or more aspects of the positive control that welds the cells of the body into a single functioning unit‐the organism as a whole…The failure in cancer is due not to any weakness of the organism but to a change in the character of the cells rendering them in one way or another insusceptible to the normal control. This statement is self‐evident when we consider the phenomena of metastasis and experimental transplantation…*.*”* ^48^

Despite the fundamental knowledge that viruses cause cancer, in 1955's/1960's, the public was allowed to consume virus‐contaminated polio vaccines. This intellectually criminal act by decision makers sharply increased cancer incidence, mortality, and morbidity of baby boomers and the subsequent generations (see below). It should be noted that prior to vaccination of public with virus‐contaminated polio vaccines, decision makers minimized, downplayed, ignored, and harassed a highly competent and concerned microbiologist (Bernice Eddy) at NIH who discovered that the polio vaccines had live and filterable viruses (eg, Simian virus, SV‐40) and predicted that contaminated polio vaccines could cause cancer epidemic.^1^, ^5^, ^8^, ^17^

The loss of too many lives and numerous polio vaccine injuries resulted in lawsuits against NIH and DHHS and resignation of directors of NIH and DHHS, constituting little more than a slap on the hand!.^1^ Despite this record, the power of the medical establishment over exclusive decision‐making and over public health in general increased to its current scary level. In the last few decades induction of several infective respiratory diseases such as Swine flu, SARS or MERS, Zika, and the current pandemic on coronavirus (Covid‐ 19) that resulted in global lockdown, the crash of the economy, scare tactics and heavy publicity, debates, controversies for masking, treating and marketing vaccines on a global scale that are parroted by major media have created serious scientific/medical and legal concerns about future of public health internationally^81^, ^83^, ^86^, ^87^ (manuscript in preparation).****’††††

The basis for the emergence of increased risk of pathogenic and retrovirus infections (eg, flu, HIV) or SARS, MERS, and coronavirus that created an urgent need for developing pathogen‐specific vaccines initiated questions on the potential presence of live pathogens (similar to SV‐40) in the media that vaccines were prepared and consumed by the public in the past three decades^1^, ^20^ (manuscript in preparation)‡‡‡‡

RETRACTED

### 3.2 Ignoring while abusing evidence for link between inflammation and tumorigenesis and angiogenesis

*It is dangerous to be right, when the government is wrong*. Voltaire

Epidemiological reports on circumstantial evidence for an association between sites of prior injuries/chronic irritation or inflammation and the increased risk of cancer have been documented for a century.^1^, ^5^, ^8^, ^10^, ^41^, ^44^, ^45^, ^46^, ^47^, ^49^, ^50^, ^51^, ^52^ In few such articles, professionals noted major gaps on direct evidence for a link between inflammation and induction of carcinogenesis and angiogenesis. Biological gaps were also noted on evidence for identifiable stages of immune alterations toward tumorigenesis or cancer. The cancer establishment has continued ignoring these important biological gaps on the initiation events that lead to immune dysfunction toward tumorigenesis and angiogenesis.

Since 1998, analyses of data on our original studies that were conducted on experimental models of acute and chronic ocular inflammatory diseases, unexpectedly demonstrated a series of evidence that satisfied at least two of the major knowledge gaps on the role of inflammation in cancer immunobiology^1^, ^5^, ^8^, ^20^, ^25^, ^26^, ^41^, ^42^, ^43^, ^44^, ^45^, ^46^, ^47^, ^49^, ^50^, ^51^, ^52^ (Figure 2):

- Evidence on direct association between inflammation and induction of tumorigenesis and angiogenesis;
- Time course kinetics of inflammation‐induced at least three identifiable phases of immune dysfunction toward multistep tumorigenesis;
- In 2014, further analyses of original data also revealed the first evidence on sequential interactions and synergies between activated host and recruiting immune and non‐immune cells in the direction of tumor growth. These data also incorporate the missing evidence on immune disruptor‐induced initial events in altering immune responses.^42^

### 3.3 Author's accidental discoveries: Initiation events in tumorigenesis and angiogenesis‐ Direct evidence for a link between inflammation in multistep immune dysfunction. Intellectual challenges at NCI/NIH since 1998 (Intellectual Me Too!)

Since 1998 at NCI/NIH, Khatami followed the logical, careful, and integrated approaches of Burnet that led him to the theory of immune surveillance. Analyses of original data that the author's team established at the University of Pennsylvania on experimental models of ocular acute and chronic inflammatory diseases in 1980s, led her to a series of reports that were suggestive of the first and only series of data on direct association between inflammation (initiation events) and multistep tumorigenesis and angiogenesis.^1^, ^5^, ^8^, ^20^, ^41^, ^42^, ^43^, ^44^, ^45^, ^46^, ^47^, ^50^ Further analyses and integration of data in the fields of immunology‐inflammation, cancer, and developmental biology, aging, biomarkers, molecular diagnosis and therapeutics led to recent definitions of inflammation for maintenance of health or induction of diseases. A number of concepts and comprehensive proposals were submitted in an effort to promote the role of inflammation in cancer research for early molecular diagnosis, design of clinical trials, use of patients’ biospecimen, and potential agents (eg, SH‐containing agents, captopril, Sulindac, aspirin) for cancer chemoprevention. Khatami also developed a working project, standardizing cancer biomarkers criteria for developing effective databases for oncology research, using an inflammatory mediator (M‐CSF), as a prototype to tailor and test the sensitivity and specificity of M‐CSF, in comparison with conventional mediators (NCI‐Invention, Fed. Reg, 2005).^1^, ^5^, ^8^, ^10^, ^20^, ^41^, ^42^, ^52^

Decision makers and their handlers at NCI/NIH, severely opposed, ignored, denied, minimized, and rejected the submitted concepts and comprehensive proposals on the important role of inflammation in cancer research and therapy. However, in the last two decades, it seems that Khatami's challenging efforts awakened the entire cancer community around the world. Members of the establishment fragmented the submitted ideas and used them as a front for collecting more funding from the cancer‐stricken public. Significant increased funded projects focus on isolated numerous cellular and molecular aspects of inflammation‐immunity for cancer research and therapy; using site‐specific tumor models, expensive specific technologies, and related networks. However, the reductionist approaches on the topic of inflammation created further confusion and ongoing debates on what inflammation does, whether it prevents cancer or it causes cancer,^1^, ^5^, ^8^, ^20^, ^51^ (NCI/NIH scientific and legal documents, since 1998).

RETRACTED

It is noteworthy that current literature in the field is flooded with hundreds of thousands of articles on the structures and substructures of numerous pathogens, their roles in experimental models of diseases; or numerous identified genetic mutations in cancer molecular tsunami to use specific expensive technologies for research, diagnosis or treatment and pathogen‐specific vaccine technologies. However, peculiarly, except for our accidental discoveries that were established in 1980s, very little is known about how stimuli (immune disruptors, pathogens) systematically would induce initiation processes in altering immune response dynamics toward time‐dependent multistage disease development.

## 4 INTELLECTUAL IGNORANCE THAT ABNORMAL GENE MUTATIONS IN CARCINOGENESIS ARE CONSEQUENCES OF SEVERELY DISTURBED IMMUNITY. IDENTIFYING ENDLESS MUTATIONS IN RESEARCH AND DRUG DEVELOPMENT THAT FAILED PATIENTS

*The truth is incontrovertible; malice may attack it, ignorance may deride it, but in the end, there it is*. Winston Churchill

Advances in technologies for identification and sequencing of genetic mutations and over‐ or under‐expression of gene products provide evidence that individual patients have different average rates of evolving mutations during examination and growth patterns of cancer mass. For example, patients with lung cancer demonstrate 200‐300 mutations per tumor, while patients with esophageal or colon cancer present 50‐100 DNA mutations per tumor.^1^, ^5^, ^8^, ^11^, ^20^, ^49^ The Cancer Genome Atlas (an NCI‐funded project) identified thousands of gene mutations in too many site‐specific cancers. Over 30,000 gene mutations are reported in breast cancer tissue alone.^1^, ^11^, ^54^ The mutations that are identified in cancer molecular tsunami for the purpose of drug development and claims of “targeted” therapy, “precision,” or “personalized” medicine, or recently fashionable ‘immunotherapy’ have repeatedly failed patients. Abnormal or excessive activation or deactivation of genomic pathways (eg, chromosomal, DNA/ RNA, hypo‐, hyper‐methylation and epigenomic modifications) and associated expression and co‐expression of tumoricidal or tumorigenic mediators, receptors and decoy molecules, enzymes/proteins/growth factors (eg, TNFRs, ILs, IRAK‐M, SODs, mTOR, FGF, MMPs, cMyc) are the results of overstimulation (exhaustion) of molecular components of the synchronized immune response dynamics; loss of electrobiology and skewed balance between tumoricidal (apoptosis, Yin or degeneration) and tumorigenic (wound healing, Yang, or regeneration) properties of immunity. The evolving mutational patterns and the number of mutations at specific cancer sites (cancer molecular tsunami) make such expensive projects, intellectually deceptive, worthless, and irresponsible and they are “scientific/medical Ponzi schemes.”^1^, ^5^, ^8^, ^10^, ^11^, ^49^, ^50^, ^51^

Decision makers of such ill‐conceived and dangerous therapeutic projects who often use a combination of chemotherapy with whole or partial body radiation, totally disregard the important molecular compensatory mechanisms of immune responses toward inhibitors of apoptotic factors (eg, monoclonal antibodies, growth factors‐kinases inhibitors) against specific factors, enzymes or receptor molecules.^1^, ^5^, ^8^, ^20^ Other failed clinical trials include the use of hormone replacement therapy; finasteride (synthetic 4‐azasteroid) to inhibit type II‐5‐α‐reductase that converts androgen testosterone to 5‐α‐dihydrotestosterone; PSA measurement for prostate cancer therapy and diagnosis.^1^, ^5^, ^8^, ^10^, ^11^, ^12^ §§§§ Such therapies in an already immune‐compromised patient often induce immune tsunami (cytokine storm) in tissues/organs and lead to relapse, fatigue, cachexia, sarcopenia, thromboembolism, multiple organ failures (MOFs), and death.^1^, ^8^, ^10^, ^11^, ^20^

The quality of blood (eg, fresh/young, frozen or old and storage procedures, using preservatives and duration of blood storage) that are employed for transfusion or iron supplementation in therapy‐induced anemia is also among factors that are often ignored or not reported in the literature. There are considerable differences in the outcomes of such procedures (eg, iron toxicities, “storage lessions,” infections, complications with bleeding and thrombocytopenia, compatibility, age, and immune status of donor or recipient),^55^, ^56^ (manuscript in preparation).

RETRACTED

## 5 AUTHOR'S SUMMARY OF ACCIDENTAL DISCOVERIES‐MULTISTEP IMMUNE DYSFUNCTION: SETTING STAGE FOR VACCINE‐INDUCED INJURIES

*It is better to deserve a prize and not have it, than to have a prize and not deserve it*. Mark Twain

Summary results of a series of our original studies and recent analyses of data are relevant when toxicities of vaccines and adjuvants are discussed. Guinea pig eyes were repeatedly stimulated and challenged with topical administration of FLOA (immune disruptor, antigen) with or without infective agents (A. Summ, parasite and extracts), adjuvants (pertussis), tumor‐promoting agents (TPAs) for up to 30 months. Major clinical, histopathological, and immunological findings and observations are summarized below^1^, ^5^, ^8^, ^20^, ^41^, ^42^, ^43^, ^44^, ^45^, ^46^, ^47^, ^50^, ^51^, ^52^:

- **Acute/Immediate, Self‐Terminating Responses** (within 2 weeks of tissue sensitization/stimulation with antigen/stimulus): clinical strong or weak reactions associated with varying degrees of tissue edema, tearing, scratching and vascular hyperpermeability, induction of IgE antibody synthesis, release of histamine and prostaglandin (PGF‐1α) as first and secondary mediators;
- **Intermediate Phase (Down‐Regulation Phenomenon)** (within couple of mons of repeated stimulation of CALTs): clinical desensitization, heavy infiltration of eosinophils into epithelium, goblet/mucus secreting cells and ocular secretion;
- **Chronic Phase** (within 30 mons of tissue stimulation): induction of tumor‐like lesions, extensive angiogenesis, massive hyperplasia of lymphoid tissues (upper and lower bulbar conjunctiva, activation of macrophages, impaired boundary of lymphoid tissue and infiltration of different size lymphocytes into epithelial tissues, follicular formation, epithelial thickening and/or thinning (necrosis or growth often noted in the same tissue sections), increased MCs degranulation (‘leaky’ MCs), histiocytes (DCs) and lymphatic channel activations;
- **Newborn Sensitivity toward Antigen Challenge**: Preliminary observations demonstrated that newborn guinea pig eyes, born from sensitized parents responded to 1^st^ or 2^nd^ challenge by antigen, suggesting predisposition of fetus/unborn tissues, involving B/plasma cells and MCs sensitization/activation, through parental sensitization. These observations suggest that parental sensitization induced genetic mutations and increased (induced) allergies (inheritance, congenital or neonatal?) in unborn and newborn animals;
- **Local and Distal Tissue Sensitization**: Animals with strong ocular responses often presented wheezing‐like reactions, suggesting sensitization and activation of lung mast cells (preliminary observations);
- **Mixture of Antigen with TPAs**: Mixing antigen with tumor promoting agents (TPAs, phorbol esters) shifted induction of tumorigenesis‐ hyperplasia to earlier time‐frames (within 6 months) suggesting activation of kinases (preliminary observations)*****.

RETRACTED

Extension and confirmation of these accidental discoveries and observations are among projects that perhaps deserve taxpayers’ investment. Outcomes are expected to provide insightful understanding of short‐ or long‐term effects of oxidative stress, or toxicities of drugs and vaccines during pregnancy and after birth in induction of diverse immune disorders^1^, ^5^, ^20^, ^58^ (Figures 1 and 2) (see below).

### 5.1 Recent Definitions of Effective Immunity: Yin and Yang of Acute Inflammation: Vaccine‐Induced Injuries or Destruction of Natural Biorhythms

Definitions of acute and chronic inflammation (Yin‐Yang) was first reported in 2008^43^ and further extended since then.^1^, ^5^, ^8^, ^20^, ^24^, ^42^, ^43^, ^44^, ^47^, ^50^, ^51^ Effective immunity was defined as the balance between two highly regulated and biologically opposing arms, termed the Yin (pro‐inflammatory, apoptosis, tumoricidal, degeneration) and the Yang (post‐inflammatory, growth promoting, wound healing, tumorigenic, regeneration) of self‐terminating properties of acute inflammation with dual or biphasic roles. Protective mechanisms of acute inflammation involve amazingly precise electro‐molecular (bioelectrical) signal transduction communications that are synchronized (time‐dependent electro chemical control switches with circadian behaviors) or autonomic sympathetic and parasympathetic activities between immune and non‐immune systems, involving innate and adoptive immune cells and vascular‐metabolic‐neuronal‐hormonal/endocrine‐lipids/adipocytes; or cell mediated and humoral immunity (CMI, HI).

RETRACTED

Self‐terminating properties of acute inflammation requires differential energy expenditure from mitochondrial oxidative phosphorylation (burst of energy, ATP hydrolysis) during Yin events; and low energy (ATP hydrolysis) from glycolysis (glucose metabolism) during Yang events. Dual processes in Yin‐Yang events would allow mitochondrial recovery and biosynthesis of TCA intermediates. Depending on the nature and potency of stimuli and susceptibility or type of host tissue (eg, immune‐responsive or immune‐privileged), Yin events involve generation of precise quantities of danger molecules, pro‐inflammatory cytokines/chemokines, oxidants and enzymes [eg, TLRs, vasoactive agents (histamine), NO, TNFα, PGs, neurotoxins, ILs, ROS, caspases/oxidases] from activated cells for the purpose of destroying internal or external foreign entities and injured host tissues. Immediately following Yin events, phenotypes of activated immune and non‐immune system with dual properties provide specific signals to express mediators with reducing or anti‐inflammatory properties for resolving inflammation and repairing, reconstructing or remodeling the injured host tissue. Yang pathways include expression of decoy receptor molecules, antioxidants, growth factors, hormones, enzymes and cytokines (eg, ILdRs, superoxide dismutases (SODs), kinases, IRAKM, TNFdRs, INFs, FGF, VEGF).^1^, ^5^, ^8^, ^20^, ^24^, ^43^, ^44^, ^51^, ^52^

In general, the molecular/cellular components that make‐up the highly synchronized and controlled signal transduction mechanisms of effective immunity (CMI or HI), play dual roles during an inflammatory condition. For example, stimuli would induce activation of macrophages (MΦs, M1/tumoricidal and M2/tumorigenic phenotypes) or other antigen presenting cells (APCs). M1 phenotypes induce appropriate and often simultaneous electrochemical signals to express receptors/danger molecules, surface proinflammatory mediators, and activate T and B cells, vasculature, mucus‐secreting cells, as well as activation of metabolic and neuronal pathways. Major outcomes of stimuli‐induced activation of cells are burst of energy (ATP hydrolysis) from mitochondria (oxidative phosphorylation) accompanied by release of ROS and numerous other tumoricidal (Yin) mediators, to destroy unwanted agents and infected/injured host tissue. Following destruction of stimuli, simultaneously M2 and their counterparts in T (eg,Treg) and B cells, vasculature and metabolic‐neuronal systems, signal for shutdown/resting status of mitochondria (allowing regeneration of TCA cycle), and expression of tumorigenic (post‐inflammatory) mediators (Yang) to terminate and resolve inflammation, and to repair host tissue.

RETRACTED

Oxidative stress or unresolved (subclinical) inflammation or continuous stimulation of tissues was proposed, as a common denominator in initiation and progression of nearly all chronic diseases (eg, asthma, emphysema, hypertension, gastritis, colitis, thyroiditis, prostitis, atherosclerosis, multiple sclerosis, ALS, lupus, Alzheimer's, Parkinson's, obesity, adult‐ onset diabetes and cardiovascular complications, stroke and site‐specific cancers) that are often features of age‐associated illnesses.^1^, ^5^, ^8^, ^20^, ^42^, ^43^, ^44^, ^49^, ^51^, ^52^, ^53^

Author's original concept on definitions of Yin and Yang properties of effective immunity seems to serve larger applications, than originally proposed, for understanding of the complex biphasic and synchronized activities of system biology (autonomic sympathetic and parasympathetic neuronal system) for maintenance of health or initiation of diseases.^1^, ^5^, ^20^

Analyses and integration of a wide range of data on infections, drugs and vaccine‐related topics support a hypothesis that frequent infections, irritations and vaccination with pathogen‐specific vaccines and incipient, cause overstimulation (exhaustion) of mitochondria that would adversely influence the electrobiology of immune response profiles (Yin‐Yang) and pose diverse health consequences in young and old, particularly in the unborn, newborn, infant or immune‐compromised individuals (see below)^1^, ^5^, ^8^, ^20^, ^23^, ^24^, ^43^, ^44^, ^47^, ^49^, ^78^, ^79^, ^80^, ^81^, ^82^, ^83^, ^84^, ^85^ (Figures 1, 2, 3).

**FIGURE 3:** Schematic representation of toxicities of vaccines altering fetus growth and development and bases for immediate or long‐term immune disorders, at different stages of life. The complex scheme represents that current pathogen‐specific vaccines (MMR, Hep, Flu, dTab, HPV, meningitis) and adjuvants [Al, Hg, detergents, solvents growth factors (PS80, Silica A, fetal serum)] would alter immune electromagnetic response profiles in tissues and damage differential bioenergetics of mitochondrial oxidative phosphorylation, leading to diverse immune disorders. It also depicts that vaccination of unborn/newborn and infants lead to shifted disease categories (congenital, hereditary, neonatal or induced) to increase the induced diseases (black box). See text

RETRACTED

### 5.2 Development of mitochondria and effective immunity [Yin‐Yang] after birth: Thermodynamic laws of open access system in growth and development: A hypothesis

Recently, we theorized that mitochondria and Yin arm of immunity are fully developed/functional after birth; when the newborn is exposed to atmospheric oxygen pressure and for completion of organ development; during which infant becomes independent from mother's immunity (within 2 years after birth). After birth and throughout adulthood and aging, the human body requires an effective immunity to combat diseases. The multi‐cellular complex signal communications of effective immunity require differential energy‐demand processes for tear (degeneration, Yin) and wear (regeneration, Yang) to effectively defend and maintain individual health (power within) against all elements that are perceived threatening body's survival (power without)^1^, ^5^, ^20^, ^24^ (manuscript in preparation).

In a working model in an attempt to explain the complex electrobioloy and differential roles of mitochondria in autonomic neuronal sympathetic‐parasympathetic or on‐off signal switches of effective immunity, the author theorized that the law of thermodynamics of open systems would apply, in varying degrees, to the growth patterns of human biology; from orderly growth and development of fetus, to adulthood, aging and disease processes.^5^, ^20^ During fetus growth, except for those events that are required for organogenesis and angiogenesis, occurring under low/limited oxygen pressure of protective environment of placenta, Yin arm of immunity and mitochondria are not fully developed and not required. Otherwise, oxidative stress and expression of apoptotic factors could result in fetus abortion, preterm birth, low growth rate (low weight at birth), retardation or defects in fetus organ development or childhood cancers.^5^, ^20^ As detailed below, a potential factor in reported increased in childhood diseases or cancers or SIDs are presence of oxidative stress‐ (eg, vaccination of pregnant woman) and expression of exaggerated wound healing or apoptotic factors that are likely to alter/skew expression of constituent vs. induced receptors and adversely affect growth of newborn, immediately after birth or later on during adulthood or aging process^1^, ^5^, ^20^ (manuscript in preparation)] (Figures 1 and 3).

Immunologically, one may argue that exposure of unborn, newborn and infant to even ‘safe vaccines’ or other biologics (stimuli) could retard‐impair and threaten proper development of mitochondria and tissues/organs (eg, lung, kidneys, liver, brain, reproductive system) causing immediate‐short‐, or long‐term health consequences. As shown below, pathogen‐specific vaccines (eg, polio, swine flu, hepatitis a, b, c, MMRs, meningitis, shingles, anthrax, pertussis, HPV, SARS, Ebola, Zika, or ‘covid‐19’) and incipient weaken/destroy the complex electrobiology of immunity and **Not Promote It**!.^1^, ^5^, ^8^, ^11^, ^17^, ^20^, ^27^, ^28^, ^29^, ^30^, ^31^, ^32^, ^33^, ^34^, ^35^, ^36^, ^37^, ^38^, ^39^, ^40^, ^41^, ^42^, ^43^, ^44^, ^45^, ^46^, ^47^, ^48^, ^49^, ^50^, ^51^, ^52^, ^53^, ^54^, ^55^, ^56^, ^57^, ^58^, ^59^, ^60^, ^61^, ^62^, ^63^, ^64^, ^65^, ^66^, ^67^, ^68^, ^69^, ^70^, ^71^, ^72^, ^73^, ^74^, ^75^, ^76^, ^77^, ^78^, ^79^, ^80^, ^81^, ^82^, ^83^, ^84^, ^85^, ^86^, ^87^, ^88^, ^89^, ^90^, ^91^, ^92^, ^93^, ^94^, ^95^, ^96^, ^97^, ^98^, ^99^, ^100^, ^101^, ^102^, ^103^, ^104^, ^105^, ^106^, ^107^, ^108^, ^109^, ^110^, ^111^, ^112^, ^113^, ^114^, ^115^, ^116^, ^117^, ^118^, ^119^, ^120^, ^121^, ^122^, ^123^, ^124^, ^125^, ^126^, ^127^, ^128^, ^129^, ^130^, ^131^, ^132^, ^133^, ^134^, ^135^, ^136^, ^137^, ^138^, ^139^, ^140^, ^141^, ^142^, ^143^, ^144^, ^145^, ^146^, ^147^, ^148^, ^149^, ^150^, ^151^, ^152^, ^153^, ^154^, ^155^, ^156^, ^157^, ^158^, ^159^, ^160^, ^161^, ^162^, ^163^, ^164^, ^165^, ^166^, ^167^, ^168^, ^169^, ^170^, ^171^, ^172^, ^173^, ^174^, ^175^, ^176^, ^177^, ^178^

RETRACTED

### 5.3 Low energy consuming arm of immunity from glycolysis (Yang): Vaccination during pregnancy disturb delicate biology of trophoblast‐placenta and orderly fetus growth. Hypothesis

Orderly growth of fetus or disorderly growth of cancer masses requires low energy consumption from glycolysis (Warburg effect); where growth processes occur under low oxygen tension. The orderly growth of fetal mass was suggested to be peculiarly comparable to the disorderly growth of cancer cells having undeveloped or dysfunctional mitochondria, respectively.^1^, ^5^

In brief, after birth the dual capacity of effective immunity (Yin‐tumoricidal v. Yang‐tumorigenic) and mitochondrial function are required for differential energy consumption and time‐dependent electrochemical signals (synchronized on/off switches) for maintenance of health. Protection of complex electrobiology of immunity (immune neuroplasticity) that parallels neuronal behaviors (autonomic sympathetic and parasympathetic) is the most important aspect of human health and well being.

## 6 VACCINE SCIENCES: CURRENT IMMUNOLOGICAL SAFETY CONCERNS

*Be a yardstick of quality. Some people aren't used to an environment where excellence is expected*. Steve Jobs

The concept of vaccination, or rather immunization, for protecting, promoting and defending individual health against viruses, bacteria or parasites developed in the eighteenth century, well before the important theory of immune surveillance was developed, and before better hygiene or antibiotics improved public health and reduced many preventable infectious diseases and increased longevity. The concept of protecting public health by immunization also existed before Rockefeller patent medicine and Gates patent vaccines invested a great deal in medical education to influence promotion of drug sale and to vaccinate the public with pathogen‐specific vaccines in toxic media and associated debates and controversies.^1^, ^2^, ^4^, ^5^, ^12^, ^13^, ^17^, ^18^, ^20^, ^21^, ^22^, ^23^, ^24^, ^28^, ^30^, ^31^, ^32^, ^33^, ^36^, ^37^, ^38^, ^39^, ^40^, ^59^, ^60^, ^61^, ^62^, ^63^, ^66^, ^67^, ^68^, ^70^, ^73^, ^77^, ^83^, ^93^, ^94^, ^96^, ^97^, ^110^, ^111^, ^116^, ^128^, ^136^, ^137^, ^138^, ^139^, ^140^, ^141^, ^142^, ^143^, ^144^, ^146^, ^147^, ^148^, ^149^, ^150^, ^156^, ^158^, ^160^, ^161^, ^162^, ^163^, ^164^, ^165^, ^166^, ^168^, ^169^, ^170^, ^171^, ^172^, ^174^, ^175^, ^181^, ^189^, ^190^, ^191^, ^192^, ^193^, ^194^, ^195^, ^196^, ^197^, ^205^, ^206^, ^212^

Seven/eight decades ago, vaccines were considered relatively safe and effective in promoting/boosting immunity and preventing diseases when healthy children (2 years or older) were vaccinated with few dead/inactivated pathogens (eg, measles, mumps, diphtheria, smallpox) that were prepared in saline solutions. The overall review of data on epidemiological studies and/or comparison of vaccinated and unvaccinated children at different settings around the globe, despite variations in methods and procedures, suggest that natural exposures to infective agents (eg, measles and mumps) are associated with lower rates of mortality from chronic diseases such as atherosclerotic and cardiovascular diseases^31^, ^174^ †††††.

RETRACTED

In general, outcomes of an acute inflammation (eg, responses to infective agents) are lymphocyte‐derived clonal expansion, increased synthesis of pathogen‐(or allergen) specific antibodies and memory cells.^1^, ^5^, ^8^, ^12^, ^20^, ^24^, ^25^, ^41^, ^42^, ^43^, ^44^, ^45^, ^46^, ^47^, ^49^, ^50^, ^51^, ^52^ Synthesis of antibodies (eg, IgGs, IgE, IgA, IgM) and memory cells (B/plasma or T cells) are needed for priming the immune system (boosting immunity). Upon next exposure to similarly structured infective agents, the host's primed immune system unleashes appropriate and precise quantities of required neutralizing antibodies and pro‐, and anti‐inflammatory mediators [eg, TLRs, vasoactive agents (histamine), cytokines, oxidants, enzymes, neurotoxins or growth factors and antioxidants] to destroy pathogens and injured/infected tissues and also to repair and remodel infected host tissues (see above). Therefore, occasional exposures of healthy children to infective agents are expected to boost natural immunity and prevent many diseases throughout life.^1^, ^5^, ^8^, ^20^ Even occasional exposure of healthy adults to potent pathogens (eg, meningococcal, coronavirus) is likely to protect the body from cardiovascular and respiratory diseases or cancer, if the victims successfully survive pathogen‐induced cytokine storms (immune tsunami or exaggerated immune responses) that are expressed against such pathogens,^1^, ^5^, ^20^, ^24^ (unpublished observations).

In brief, it takes approximately 2 years for newborn‐infant to be immunologically independent from mother's immunity. Newborn's exposure to oxygen pressure and parallel completions of mitochondria and organ development and Yin (tumoricidal) arm of immunity provide the growing baby the required natural protection (defending capacity, power within) against external and internal foreign elements for maintenance of health.^1^, ^5^ We also proposed that after birth, the Yin arm of effective immunity is required for metabolism of essential branched amino acids (eg, val, leu, isoleu) for protein biosynthesis and structural integrities of tissues and mitochondrial function.^1^, ^5^, ^20^

## 7 VACCINE TOXICITIES: RETARDATION OF MITOCHONDRIA AND IMMUNE RESPONSE PROFILES. SEEDS OF IMMUNE DESTRUCTION AND INDUCTION OF MILD, MODERATE OR SEVERE IMMUNE DISORDERS IN UNBORN, NEWBORN, INFANT, CHILDREN AND ADULTS

As noted above, the current emphasis to frequently vaccinate public with pathogen‐specific vaccines that are prepared in toxic incipient/media are likely the major factors in causes, exacerbation and consequences of impaired (retarded) mitochondrial function and Yin (tumoricidal) capacities of effective immunity in reported increased disease status in young and old in America. Stimuli (vaccines)‐induced oxidative stress and suppression of immunity are likely the major risk factors in significant increase in allergies and other immune disorders (eg, asthma, autism, tics and Tourette's syndrome, hot flashes, fatigue, epilepsy, vasculitis, urticaria, pancreatitis, obesity, type I or II diabetes and cardiovascular complications, anemia, stroke, encephalitis and other neurodegenerative and autoimmune diseases or cancers) and impaired (lowered) fertility rates in younger generations in America^1^, ^5^, ^8^, ^12^, ^13^, ^14^, ^17^, ^19^, ^20^, ^21^, ^22^, ^24^, ^28^, ^29^, ^30^, ^31^, ^32^, ^33^, ^34^, ^36^, ^37^, ^38^, ^39^, ^40^, ^49^, ^50^, ^51^, ^52^, ^53^, ^57^, ^116^, ^117^, ^176^, ^192^, ^220^ (Figures 3 and 4).

RETRACTED

**FIGURE 4:** Schematic representation of toxicities of vaccines and incipient in altering mitochondrial function and diverse activities of histidine‐histamine pathways toward increased induction of diseases. Vaccine incipient/excipient (eg, metals, growth factors, DNA/RNA, and fetal tissues) are depicted to alter immune‐neuronal response dynamics, influencing genomic, mitochondrial, metabolic, and physiological functions of gastric secretion, energy levels (ATP/ADP), cell cycle and brain activities as well as vasculature, tissue growth or necrosis. The scheme depicts that 140–200 genes are involved in histamine‐histidine metabolic‐neuro‐immune pathways. Altered tissue bioenergetics is depicted to cause induction of mild, moderate, or severe immune disorders (black box). The scheme also represents that current vaccines shift the incidence of all classically known diseases (congenital, hereditary, neonatal, or induced) to increase the level of induced diseases. See text

### 7.1 Debates and controversies on reported safety of vaccines and incipient

Analyses of data on vaccines and the impact on health of the unborn/neonatal, newborn and infant include review of documents on regulatory governmental agencies (eg, FDA, CDC, WHO), Public Health Informatics Network, American Medical Informatics Association, National Animal Health Management Emergency Management System and USDA, information on funding support from government, industry and ‘philanthropists’ to study and promote vaccines, manufacturers’ inserts on vaccines contraindications, reports on spontaneous electronic adverse events on cancer drugs and vaccines, websites and blogs as well as, congressional debates, legal and financial incentives to professionals for promoting and publicizing vaccines, experts depositions in vaccine injury courts and awards to vaccine injured individuals^1^, ^5^, ^18^, ^64^, ^77^, ^94^, ^136^, ^137^, ^140^, ^141^, ^142^, ^143^, ^144^, ^169^, ^172^, ^175^, ^176^, ^177^, ^178^, ^179^ ‡‡‡‡‡’§§§§§ ^,^ ****** ^’^ †††††† ^’^ ‡‡‡‡‡‡.

Unfortunately, governmental guidelines, particularly on cancer or vaccine‐related statistics, safety procedures, vaccine effectiveness or reported injuries are provided on behalf of medical establishment with little independent evaluation, considerations or validation of biological sciences, medical ethics and conflicts of interest, or safety considerations. The official guidelines by governmental agencies are skewed, biased and often laced with deception and cover ups on disease causes (eg, SIDS, vaccine injuries, drug toxicities, clinical trials on exclusion/inclusion criteria). Often official information is not worthy of serious considerations once the scientific pros and cons are weighed, particularly regarding information on root causes of cancer epidemics, over‐, under‐diagnosis of diseases, toxicities of drugs, biologics or vaccines safety^1^, ^2^, ^3^, ^4^, ^5^, ^6^, ^7^, ^8^, ^9^, ^10^, ^17^, ^20^, ^21^, ^22^, ^23^, ^50^, ^51^, ^52^, ^64^, ^69^, ^71^, ^93^, ^136^, ^137^, ^140^, ^141^, ^157^, ^164^, ^177^, ^192^ §§§§§§ ^,^ ******* ^,^ ††††††† ^,^ ‡‡‡‡‡‡‡ ^,^ §§§§§§§. Often, credible scientific information that is prepared by scientists who work in the government or academia are ignored, dismissed or abused when members of the establishment decide to publicize drugs or vaccines of their choice.^1^, ^2^, ^3^, ^4^, ^5^, ^6^, ^7^, ^8^, ^10^, ^11^, ^12^, ^13^, ^17^, ^18^, ^34^, ^36^, ^37^, ^38^, ^39^, ^64^, ^69^, ^71^, ^77^, ^94^, ^143^, ^149^, ^169^, ^172^, ^176^, ^178^, ^180^, ^181^, ^182^, ^183^, ^184^, ^186^, ^187^, ^188^, ^189^, ^190^, ^191^, ^192^, ^193^, ^194^, ^195^, ^196^, ^197^

In general, diversities and extent of immune disorders [acute inflammatory responses, delayed hypersensitivity reactions, mild (subclinical inflammation, oxidative stress), moderate or severe diseases] that occur immediately after vaccination or within few days‐weeks‐ months or years later, depend on several interdependent factors as outlined below (Figures 1, 2, 3, 4):

- Age of vaccinated individual;
- Health status of vaccinated individual;
- Dosage, frequency and rout of vaccination;
- Period between subsequent vaccination;
- Composition of media/adjuvants (incipient) in vaccines;
- Nature (quality/composition, potency) of pathogenic particles in vaccines;
- Quality control (placebo) status of vaccines, procedures and standard tests for safety before public consumption;
- Quality of clinical trials (eg, inclusion or exclusion criteria, crossover trials and safety recommendations and approval of vaccines);
- Time course on reported vaccine injuries and follow up on inclusion of VAERS;

Flu shot ingredients, given to pregnant women could disturb the intricate biological networks of trophoblast‐embryo‐fetus‐placenta that are required for orderly growth of fetus. Under incomplete mitochondrial development and hypoxic conditions of placenta, organogenesis and angiogenesis of embryo‐fetus require proper architectural organization and functioning of trophoblast epithelium for providing and consuming appropriate and sufficient growth factors/hormones, nutrients, enzymes, trace elements (metals) and respective constituent or induced receptor molecules. Exposure of the embryo‐fetus to flu shot and incipient, could pose serious threats to survival and health of both mother and fetus including altered nutrients in organogenesis, transition of myoblasts to myotube development, ratios of constituent/induced receptors, as potential contributors in growth retardation or growth promotion, fetus abortion or impaired health of newborn, infant, toddler, that also influence immunity during adulthood and aging process^1^, ^5^, ^8^, ^20^, ^24^, ^27^, ^28^, ^29^, ^30^, ^31^, ^32^, ^33^, ^34^, ^35^, ^36^, ^37^, ^38^, ^39^, ^40^, ^41^, ^42^, ^43^, ^44^, ^45^, ^46^, ^47^, ^48^, ^49^, ^50^, ^51^, ^52^, ^53^, ^54^, ^55^, ^56^, ^57^, ^58^, ^59^, ^60^, ^61^, ^62^, ^63^, ^64^, ^65^, ^66^, ^67^, ^68^, ^69^, ^70^, ^71^, ^72^, ^73^, ^74^, ^75^, ^76^, ^77^, ^78^, ^79^, ^80^, ^81^, ^82^, ^83^, ^84^, ^85^, ^87^, ^88^, ^89^, ^90^, ^91^, ^92^, ^93^, ^94^, ^95^, ^96^, ^97^, ^98^, ^99^, ^100^, ^101^, ^102^, ^103^, ^104^, ^105^, ^106^, ^107^, ^108^, ^109^, ^110^, ^111^, ^112^, ^113^, ^114^, ^115^, ^116^, ^117^, ^118^, ^119^, ^120^, ^121^, ^122^, ^123^, ^124^, ^125^, ^129^, ^192^ (manuscript in preparation)] (Figures 1, 3 and 4).

RETRACTED

Examples of deception that are frequently applied to the safety of drugs or vaccines are controversies on exclusion criteria or crossover practices in conducting clinical trials for obtaining approval of drugs or vaccines.^11^, ^113^, ^139^, ^140^, ^141^, ^187^, ^189^, ^190^, ^191^, ^196^, ^197^ In the majority of clinical trials, decision makers select and recruit healthy individuals for testing safety of drugs or vaccines. Any individual with minor or major illnesses are excluded. This allows manufacturers to show maximum benefits and minimum harms of tested biologics. However, even under such selective criteria, healthy participants often experience various degrees of side‐effects that may or may not be acknowledged or documented during the marketing of such drugs. Vaccine approval voting is conducted through FDA (eg, VRBPAC) or CDC (eg, ACIP) committees, whose members are often industry, government employers or grantees (principal investigators) who receive funding to study and patent drugs/vaccines and to collaborate with manufacturers for large scale development and for marketing to the general public, healthy or not.^2^, ^8^, ^18^, ^70^

An example of vaccine propaganda is found in the marketing of HPV vaccines (Gardasil or Cervarix) that were approved to target the young generation, claiming to prevent cervical cancer. Segments of papilloma virus (types 6,11,18) and recombinant DNA technologies are used in media/incipient that has combination of Al, PS80, SIO2, Saponin.^8^, ^12^, ^14^, ^19^, ^24^, ^110^, ^131^, ^132^, ^133^, ^134^, ^137^, ^138^, ^139^, ^143^ Review of related data suggest that HPV vaccines and adjuvants are associated with mild or severe adverse reactions (VAERS), including autoimmune diseases, fibromyalgia, tachycardia, ovarian failure, fatigue, without any benefits in preventing incidences of cervical and related cancers^8^, ^12^, ^14^, ^66^, ^70^, ^71^, ^108^, ^110^, ^136^, ^137^, ^138^, ^139^, ^143^ ^,^ ††††††††’‡‡‡‡‡‡‡‡. In a comprehensive review^14^ Giannotta and Giannotta described the mechanisms of adverse effects of vaccines (eg, HPV) and incipient in autonomic neuronal system and development of autism spectrum disorder (ASD), fatigue and vaccine‐induced altered behaviors of immune cells (microglial and astrocytes) in the brain and associated loss of BBB.

RETRACTED

### 7.2 Vaccines incipient (ingredient, adjuvant, excipient): Mini electric shocks and molecular sink holes in mitochondria with loss of biorhythms and induction of diseases

Inactivated (or live) pathogens in vaccines, on their own, are immunogens (stimuli or immune disruptors) and could over‐stimulate immunity. According to manufacturer's inserts, governmental or published scientific data, majority of pathogen‐specific vaccines are prepared in media containing combinations of metals, chemicals‐biological agents such as aluminum (Al, as hydroxide or phosphate salts), mercury (Hg, thimerosal), detergents, solvents or preservatives [eg, CTAB, polymyxin, neomycin, saponin, formaldehyde, silica and derivatives, solutes (sorbitol, polysorbate 80 or 20, Tween 20), glyphosate‐herbicide, octylphenol ethoxylate or octoxynol‐10 (Triton X‐100)], genetically engineered DNA/RNA, yeast extracts, fetal tissues and organ parts or fragments^12^, ^14^, ^24^, ^38^, ^67^, ^73^, ^74^, ^77^, ^94^, ^96^, ^128^, ^130^, ^131^, ^132^, ^141^, ^144^, ^148^, ^152^, ^153^, ^156^, ^165^, ^167^, ^168^ §§§§§§§§’*********. Majority of these vaccine ingredients are not natural agents and do not participate in biochemical pathways in human physiology. These ingredients are additional foreign agents that overwhelm the immune system (see below). The ingredients that are perceived as ‘natural’ [eg, fetal serum, clumps of tissue/organ or DNA particles, proteins‐peptides (eg, ovalbumin, egg proteins, serum albumin, hydrolyzed porcine gelatin), amino acids (arginine, glutamate, or L‐histidine)] could disturb physiological activities and immune responses, particularly affecting the growing embryo‐fetus (unborn/neonate), newborn and infant whose organ systems, gut microbiome composition and immunity are not fully developed, or individuals who are immune compromised^1^, ^4^, ^5^, ^8^, ^12^, ^14^, ^17^, ^31^, ^32^, ^33^, ^34^, ^35^, ^36^, ^37^, ^38^, ^39^, ^40^, ^50^, ^58^, ^61^, ^62^, ^63^, ^64^, ^66^, ^67^, ^68^, ^70^, ^71^, ^141^, ^144^, ^148^, ^152^, ^153^, ^156^, ^165^, ^167^, ^168^ (Figures 3, 4, 5).

RETRACTED

**FIGURE 5:** Schematic representation of toxicities of metals and other ingredients in pathogen‐specific vaccines in induction of mild, moderate, or severe immune disorders. Metals such as aluminum (Al) or mercury (Hg) are depicted to compete with essential trace elements and alter tissue biological activities (see blue box and center divided circle), influencing mitochondrial bioenergetics metabolism and immune response profiles in tissues. The scheme depicts that vaccines and ingredients differentially influence tissues that are immune‐privileged (brain, CNS, reproductive organs) or immune‐responsive (epithelial, endothelial, mucus, fibroblast) in the genesis of wide ranges of immune disorders (tissue necrosis or growth). See text

### 7.3 Toxicities of metals in vaccines: Mini electric shocks in mitochondria altering electrobiology of vascular‐metabolic‐neuronal‐hormonal pathways

Aluminum (Al and its salts) or mercury (Hg, thimerosal) possess inert properties in nature, with cationic capabilities (eg, Al^+3^, Hg^+2^) to interact with charged molecules and act as electronic magnets. Biologically, presence of these metals in injected vaccines could compete, scavenge (chelate) or act as cationic sinks and damage the function of essential metals and trace elements (Fe^+2^, Fe^+3^, Cu^+1^, Cu^+2^, Zn^+2^_,_ Ca^+2^, Mg^+2^, Se^+2^) that are required for a wide range of cellular functions. In general, presence of Al or Hg in vaccines is likely to interfere with required proton pumping and maintenance of differential electronic charges across cellular components. Among numerous cellular functions that are likely influenced by the presence of Al or Hg are transport and function of intra‐, extra‐cellular charged proteins, amino acids and cationic‐anionic trace elements across membranes [eg, ATP/ADP/AMP, Na^+^/K^+^ exchanger, Na^+^/H^+^ exchanger, water channels, active/passive transport of solutes, osmolytes or nutrients (eg, myo‐inositol, pyridoxal phosphate, ascorbic acid)]. Overview and integration of fragmented data on vaccine‐related topics, vaccine injuries and inflammatory/immune disorders suggest that presence of non‐functional metals in vaccines create mini‐electronic shocks or ‘molecular sink holes’ and induce biological defects in mitochondria, membranes and chromosoms, damaging the regulations of biological activities in tissues including alterations of gut microbiome profiles and neuronal behaviors (Figures 1, 3–5)^1^, ^5^, ^14^, ^36^, ^59^, ^60^, ^61^, ^62^, ^63^, ^64^, ^65^, ^66^, ^67^, ^87^, ^88^, ^89^, ^90^, ^91^, ^92^, ^93^, ^94^, ^95^, ^96^, ^97^, ^98^, ^99^, ^100^, ^101^, ^102^, ^103^, ^104^, ^105^, ^106^, ^107^, ^108^, ^109^, ^110^, ^111^, ^112^, ^113^, ^114^, ^115^, ^116^, ^117^, ^118^, ^119^, ^120^, ^121^, ^122^, ^123^, ^124^, ^125^, ^126^, ^127^, ^128^, ^129^, ^130^, ^131^, ^132^, ^133^, ^134^, ^135^, ^136^, ^137^, ^138^, ^139^, ^140^, ^141^, ^142^, ^143^, ^144^, ^145^, ^146^, ^147^, ^148^, ^149^, ^150^, ^151^, ^152^, ^153^, ^154^, ^155^, ^156^, ^157^, ^158^, ^159^, ^160^, ^161^, ^162^, ^163^, ^164^, ^165^, ^166^, ^167^, ^168^, ^169^, ^170^, ^171^, ^172^, ^173^, ^174^, ^175^, ^176^, ^177^, ^178^, ^179^, ^180^, ^181^, ^182^, ^183^, ^184^, ^185^, ^186^, ^187^, ^188^, ^189^, ^190^, ^191^, ^192^, ^193^ (manuscript in preparation)]††††††††† ^,^ ‡‡‡‡‡‡‡‡‡.

RETRACTED

For example, copper (Cu^1+^ or Cu^2+^) is an essential trace element (cation) and plays crucial roles as a cofactor in mitochondrial cytochrome C oxidase and numerous other biological activities including neuronal function, wound healing, biosynthesis of collagen and vasculature. Normally, copper ions are bound to carrier molecules and distributed via carrier proteins (‘copper chaperones’) for protecting/preventing tissue damage.^36^, ^72^, ^84^, ^85^, ^91^, ^92^, ^153^, ^183^ Excess amount of copper (free) could be detrimental to respiratory chain reactions and generation of toxic hydroxyl radicals (HO^0^) causing oxidative damage not only to mitochondria, but also other extracellular‐intracellular proteins or nucleic acids and lipids (Fenton reaction) and tissue oxido‐redox potentials.^1^, ^5^, ^14^, ^20^, ^29^, ^31^, ^32^, ^33^, ^34^, ^35^, ^36^, ^37^, ^38^, ^39^, ^53^, ^55^, ^72^, ^73^, ^78^, ^84^, ^85^, ^88^, ^89^, ^90^, ^91^, ^92^, ^155^, ^182^, ^183^ Furthermore, copper and Zn^+2^ (another trace element and antioxidant) are involved in detoxifying mitochondrial ROS and superoxide dismutase1 (SOD1) activities, regulation of Cu‐mediated production of O_2_/ROS. Related studies suggest that trace elements (Cu, zinc, Fe), influence regulations of transport of triglycerides in gastrointestinal tract and are important in the function of red blood cells and endoplasmic reticulum activities. While mechanisms of toxicities or interactions between Al or Hg and trace elements on biological pathways are not well understood, it is highly likely that tissues are sensitive to such metals in vaccines, particularly affecting tissue bioenergetics (Figures 3, 4, 5). The presence of Al or detergents in vaccines could induce retardation/overload of mitochondria, causing elevated levels of Cu^2+^ in tissues (eg, liver) that would lead to vaccine‐induced respiratory or neuronal illnesses (eg, Wilson and other mitochondrial diseases).^1^, ^29^, ^36^, ^39^, ^40^, ^48^, ^49^, ^53^, ^54^, ^55^, ^56^, ^57^, ^74^, ^75^, ^114^, ^151^, ^163^, ^183^ Injected vaccines containing Al or Hg, at various stages of pregnancy, could retard fetus growth and development involving important generation, utilization, or recycling of glutathione‐related pathways (GSH: GSSH and NAD^+^: NADH) and further altering oxido‐redox potentials and incomplete mitochondria and organ development, growth impairment, immune and mitochondrial diseases after birth.^1^, ^5^, ^90^, ^102^, ^114^, ^117^, ^118^, ^151^, ^152^, ^153^, ^154^, ^155^, ^163^, ^182^

In a detailed retrospective epidemiological study, using automated Vaccine Safety Datalink (VSD), Young et al^36^ reported that vaccines containing Hg (thimerosal) were associated with neurological developmental disorders (eg, anaphylaxis, autism, ASD, tics, attention deficit disorder, and emotional disturbances) in newborn (7 and 13 months old) perhaps, due to mitochondrial dysfunction. Evaluation of data on reported vaccine injuries (eg, fatigue, hypotonia, neuropathological episodes of epilepsy, Rett syndrome or encephalomyopathy, or cancers) suggest a range of electrochemical signal defects in the function of B/plasma cells, receptor/surface molecules that could retard and alter, among other pathways, memory B cells complexes, expression of immunoglobulins, mutations in mitochondrial complexes (I, II, III, or IV), related genetic/epigenetic modifications as contributing factors in impairing pathways of oxidative phosphorylation (mitophagy), autophagy and altered endoplasmic reticulum.^1^, ^5^, ^14^, ^90^, ^102^, ^114^, ^115^, ^116^, ^117^, ^118^, ^151^, ^152^, ^153^, ^154^, ^155^, ^163^, ^166^, ^182^, ^183^

RETRACTED

### 7.4 Presence of l‐histidine in vaccines: histamine‐histidine interface‐exchange

Histidine is a natural and essential amino acid (nutrient) and structural backbone of a variety of important proteins and enzymes with diverse biological functions. With its unique imidazole side chain, histidine plays critical roles in immune response dynamics, associated with renal, neuronal, ocular and gastrointestinal biological activities. There are up to 200 genes that mediate activities of histdine‐containing proteins, such as histidine metabolic enzymes (eg, histidine decarboxylase [HDC], amino oxidase [AO]), carrier proteins, and chelating agents of trace elements (eg, Zn). Analyses of data on PTH1 or PHT1 and histidine‐histamine homeostasis and histamine receptors in neuronal tissues (eg, brain) suggest that presence of l‐His, together with Al or Hg, in vaccines alter histidine‐histamine ratio and neuropeptide regulation, particularly affecting the developing brain of fetus or newborn.^5^, ^19^, ^20^, ^36^, ^38^, ^41^, ^67^, ^79^, ^95^, ^96^, ^105^, ^122^, ^123^, ^124^, ^125^, ^126^, ^127^, ^150^, ^176^, ^177^, ^186^, ^188^, ^194^ In addition to its role in neuronal tissues histamine (catecholamine, an alkali, a potent vasoactive agent) acts as a key element and the most versatile biogenic amine, having diverse and antagonistic properties in mammalian physiology. Histamine is synthesized by enzyme histidine decarboxylase (HDC), an enzyme present in all tissues. Histamine and its receptor molecules (HRs 1–4 and subfamilies) play diverse roles in human development, acute and chronic inflammation, acid‐base balance, digestion, mucosal activities, vascular function and permeability, neuronal activities as well as, growth of cancer mass.^1^, ^5^, ^20^, ^95^, ^124^, ^126^, ^127^, ^150^, ^199^, ^200^, ^201^, ^202^, ^203^

Results of our original studies on inflammation‐induced multistep tumorigenesis and angiogenesis led to recent hypotheses that low level release of histamine (independent from IgE‐fcR degranulation of MCs [“leaky” or exhausted MCs]) is a factor in induction of tissue/cell growth that alter immune responses, including induction of autoimmune and neurodegenerative diseases or tumorigenesis and angiogenesis.^1^, ^5^, ^8^, ^20^, ^42^, ^43^, ^44^, ^45^, ^46^, ^47^, ^49^, ^50^, ^52^

Summary of diverse biological activities that are affected by abnormal levels (deficiencies or excesses) of histidine‐histamine in tissues, including altered nutritional intake, genetic mutations in production or metabolism of histidine or histamine are provided below^1^, ^5^, ^20^, ^41^, ^42^, ^43^, ^44^, ^46^, ^79^, ^95^, ^105^, ^106^, ^109^, ^124^, ^126^, ^127^, ^128^, ^148^, ^152^, ^172^, ^176^, ^177^, ^200^, ^201^, ^202^, ^203^ (Figures 4 and 5):

- Early embryonic‐fetus growth, organogenesis‐angiogenesis;
- Vasculature, innate immune cells (eg,MCs) and neuronal activities after birth;
- DNA transcription involving Zn‐imidazole at active sites of enzymes (eg, carbonic anhydrase‐CA);
- Hymolytic and redox reactions;
- Adenosyl methionine and ATP binding site of actin;
- Hydroxylation of galactosylceramide and maintenance of myelin sheath structure;
- Thyrotropin‐releasing hormone;
- Serine esterase activities of trypsin, chymotrypsin; acetylcholinesterase and blood clotting and complement cascades;
- Food or PH‐induced gastrin release of histamine from enterochromamaffin‐like cell (ECL) and activation of HDC;
- Induction of tissue growth, tumorigenesis, angiogenesis, and cancer;

Among major histidine‐histamine‐associated diseases are histinemia, kidney disease, anemia, and cancers. Hitinemia is an inherited autosomal‐recessive metabolic disorder where lack/impaired histidase activity cause an increased level of histidine and its metabolites in blood and urine and decreased uronic acid in skin and blood or elevated levels of histaminase (diaminase) activities and related metabolites and neurotransmitters such as L‐dopamine and calcitonine.^1^, ^5^, ^20^, ^101^, ^103^, ^124^, ^185^, ^197^, ^198^, ^199^, ^200^, ^201^ Rate of histinemia was shown comparable with another inherited metabolic disorder, phenylketonuria. Histinemia is associated with defects in mild neurological disorders and slow‐down of speech. Chronic kidney disease, in contrast, is associated with low histidine levels and impaired metabolites such as histamine. Furthermore, low plasma levels of histidine are associated with a higher level of histamine (perhaps increased allergies), oxidative stress and retardation of mitochondrial energy, that also affect glomerular capillaries and filtration ability of kidneys and vascular/arterial endothelium associated with pruritus. Abnormal activation of stomach digestive enzymes/hormones (gastrin) and hypergastrinemia along with altered/increased mucosal histamine production or HDC have been suggested in hyperplasia of enterochromaffin‐like cells (ECLCs or ECL). Histidine is involved in erythropoiesis, hemoglobin biosynthesis and protection of RBC in circulation and the damaging effects of ROS.^1^, ^14^, ^17^, ^20^, ^26^, ^41^, ^42^, ^43^, ^44^, ^45^, ^46^, ^95^, ^105^, ^106^, ^109^, ^124^, ^126^, ^127^, ^128^, ^129^, ^148^, ^152^, ^172^, ^176^, ^177^, ^202^, ^203^, ^222^ Anemia is also associated with histidine deficiency and oxidative stress. The presence of Al in vaccines is likely to impair histidine metabolism, by interfering with iron‐requiring proteins including transferrin, biosynthesis of erythropoiesis and RBC or complement activation cascades and contribute to vasculature lesions (eg, vasculitis) and anemia^1^, ^5^, ^20^, ^47^, ^72^, ^75^, ^82^, ^222^ (manuscript in preparation) (Figure 4).

RETRACTED

As noted above, our preliminary studies that newborn guinea pigs, born from sensitized animals, manifested strong ocular reactions (MCs activation) upon first or second challenge with antigen, suggested parental‐fetus sensitization of MCs/plasma cells and lymphoid organs, and/or premature biosynthesis of immunoglobulins (eg IgE) that influence fetus genetic predisposition and epigenetic modifications presented as diverse altered immune responses.^1^, ^5^, ^20^

Production of lactate from glycolysis and presence of essential amino acids (Ala) and histamine are characteristics of egg embryonic growth or human placenta in the transformation of myoblast to myotube and contractile myofibroblasts during organogenesis and angiogenesis.^1^, ^20^, ^219^ Data on vaccine‐related topics and increased allergies, autism, autoimmune and neurodevelopmental disorders in children indirectly support our reported observations and recent hypotheses on the role of histamine in immune disorders or cancers.^1^, ^5^, ^8^, ^10^, ^12^, ^13^, ^14^, ^20^, ^23^, ^24^, ^36^, ^40^, ^41^, ^42^, ^43^, ^44^, ^45^, ^46^, ^47^, ^49^, ^50^, ^51^, ^52^, ^60^, ^95^, ^141^, ^185^, ^197^, ^198^, ^199^, ^200^, ^201^

It is further suggested that current vaccines could induce vascular lesions by damaging endothelial cells, MMPs, heparin sulfate enzymes, GFs, and related oxidative damage in BBB, neuronal tissues, and RBC. Impaired vascular activities and altered ratios of pro‐and anti‐angiogenic factors are likely to alter vasculature function (eg, toning, permeability and hyper‐permeability) under inflammatory conditions and significantly contribute to the genesis and progression of nearly all diseases.^1^, ^5^, ^20^

Considering that vasculature is the “tree of life”, we suggest vaccine injections alter important and diverse biological functions of these tissues as listed below^1^, ^5^, ^8^, ^20^ (Figures 1, 2, 3, 4, 5):

- Vasculogenesis is the earliest events in fetus growth and development;
- Delivery of nutrient and oxygen to the tissues, and removal of gases and waste products from the tissues; keeping in mind that mechanisms of vasculature interactions are somewhat different in immune‐privileged and immune‐responsive tissues;
- Major participant (gatekeeper) and facilitator in inflammatory responses during cellular proliferation, differentiation, and infiltration of inflammatory cells into infected/injured target tissue; contributing to both apoptosis (Yin) and wound healing (Yang) processes, under acute and chronic inflammatory conditions or carcinogenesis;

In summary, vaccine‐related oxidative stress could lay a foundation to cause, exacerbate, and be a consequence of a wide range of mild, moderate, or severe immune disorders.

While, diverse contraindications of vaccines have been observed even in healthy subjects in clinical trials (exclusion criteria!) and identified in manufacturers’ inserts, heavy publicity to vaccinate the general public overlooks the health problems when industry abuses or ignores such information and targets the general public, healthy or not!, particularly because industry has little/no liability for testing the safety of vaccines^4^, ^13^, ^17^, ^19^, ^24^, ^59^, ^60^, ^64^, ^66^, ^93^, ^145^, ^157^, ^186^, ^189^, ^190^, ^191^, ^193^, ^194^ §§§§§§§§§

## 8 ECONOMIC BURDEN OF MEDICINE: WEALTH TRANSFER FROM TAXPAYERS TO ESTABLISHMENT: PUBLIC HEALTH PURCHASED!

*“If you would be a real seeker after truth, it is necessary that at least once in your life you doubt, as far as possible, all things”*, René Descartes

Since the rise of the purchasing power of Rockefeller influenced medical education and research, it seems the era of caring for public health and safety or real ‘standard of care’ has been gradually replaced by the philosophy of how to abuse power (intellectually, politically, and financially) by chipping away natural immunity and health through the abuse of drugs and pushing of vaccines. The strong partnership between governments, industry, and venture capitalists‐‘philanthropist’ has significantly weakened the conflict of interest compliance and medical ethics in conducting taxpayers‐supported projects. The drug industry has taken increasing control over the major media and of public policymaking in Congress, as well as eliminating vaccine liabilities, and changing consent forms in hospitals for patients for receiving care.^2^, ^3^, ^4^, ^5^, ^6^, ^7^, ^8^, ^10^, ^17^, ^18^, ^64^, ^167^, ^171^, ^181^, ^187^, ^189^, ^196^, ^205^, ^206^, ^207^

According to a financial analyses of healthcare ‘The Saker Blog’, the entire medical system (together with the insurance industry) has been ultimately controlled “*by one giant oligarch… Its annual value was $3.7 trillion, amounting to 17.9% of GDP (2018). That is nearly double the average of developed Western countries…”* However, “*The enormous expense does not buy Americans any better health than the Europeans get for half the price; in fact the health outcomes are far inferior in the US. In life expectancy, the US has fallen down to 33rd place, even overtaken by Cuba…Exorbitant prices on drugs, medical treatment and health insurance are crushing consumers*…”**********

As noted above, members of scientific boards and councils or review committees (eg, NCI‐BSA or NCAB, FDA, CDC review or approval groups for voting on drugs) and staff within DHHS or policymakers often have direct or indirect financial ties with drug industry‐government‐venture capitalist “philanthropists” complex, and act as rubber stamps for approving and conducting the repeatedly failed projects that are pushed by the establishment.^1^, ^2^, ^3^, ^4^, ^5^, ^6^, ^7^, ^8^, ^9^, ^10^, ^11^, ^17^, ^18^, ^21^, ^142^, ^171^, ^180^, ^181^, ^186^, ^187^, ^189^, ^192^, ^193^, ^194^, ^196^, ^202^, ^203^, ^204^, ^207^ Independent and competent professionals are becoming seriously concerned that over the last seven decades, chronic diseases that are often features of age‐associated immune disorders including cancers are manifested in children and younger generations who require hospitalization and the consumption of drugs.

RETRACTED

Table 1 shows the rising cost of vaccines, from 2000 to 2014, to vaccinate one child.

**TABLE 1:** Cost to immunize one child in the public sector has risen by over 500% since 2000

	2000	2002	2004	2006	2008	2010	2012	2013	2014
DTaP	$46.25	$59.65	$62.05	$63.98	$63.25	$66.25	$75.00	$76.90	$76.90
Polio	$31.00	$34.64	$40.40	$43.28	$45.92	$46.96	$48.96	$49.68	$49.84
MMR	$30.16	$31.22	$32.38	$34.56	$36.52	$37.27	$38.66	$39.52	$39.82
Hib	$21.96	$28.44	$33.60	$31.74	$33.78	$34.53	$35.91	$27.99	$28.08
Hep B	$27.18	$28.11	$27.45	$27.65	$28.50	$30.75	$32.19	$32.79	$33.00
Varicella	$37.14	$40.87	$47.02	$113.80^b^	$123.00	$134.16	$144.98	$150.72	$156.68
PCV	$88.50^a^	$183.96	$203.00	$230.36	$265.76	$367.00	$408.12	$428.48	$449.76
Flu	–	–	$30.00	$69.18	$205.36^d^	$175.67	$186.44	$217.39	$280.16
Tdap	–	–	–	$30.75^c^	$30.75	$28.54	$29.59	$24.63	$30.25
MCV‐4	–	–	–	$68.00	$76.35	$79.75	$164.24	$138.72	$164.24
Hep A	–	–	–	$24.31	$24.50	$26.50	$29.50	$30.50	$32.30
Rotavirus	–	–	–	$156.00	$171.60	$167.50	$182.04	$184.30	$190.40
HPV	–	–	–	–	$301.77^e^	$288.24	$335.89	$321.47	$363.09
TOTAL^f^	$282.19	$406.89	$475.90	$893.61	$1407.06	$1483.12	$1620.15	$1711.52	$1894.52

^a^ In 2000, the PCV cost to fully vaccinate one child was for half the calendar year. The CDC contract was not in place until July 1, 2000.

^b^ In 2006, ACIP recommended two doses of varicella.

^c^ Tdap replaced Td as the adolescent booster recommended by ACIP in June 2005, to provide protection against pertussis. The cost of Td has not been included in previous years due to the absence of a CDC contract.

^d^ In 2008, ACIP recommended annual influenza vaccination for all children up to age 18. Two doses are needed the first year of vaccination and 1 dose is needed annually thereafter, for a total of 20 doses.

^e^ Beginning in 2007 the total represents the cost to fully vaccinate a female including the HPV vaccine. The HPV vaccine is also recommended for males as of late 2011.

^f^ The cost of recommended vaccines is significantly higher when combination vaccines are factored in to the total cost. This table shows only the lower cost of single vaccines.

TOTAL represents the cost to vaccinate one child with vaccines universally recommended from birth through 18 years of age using federal contract prices.

Source: Centers for Disease Control and Prevention.

Association of State and Territorial Health Officials (ASTHO), March 2015.

## 9 WORTHINESS OF CURRENT SCIENTIFIC PUBLICATIONS ON CANCER AND VACCINE SCIENCES: WHEN GOVERNMENTS‐POLITICIANS‐DISEASE INVESTORS (PHILANTHROPISTS) DECIDE ON PUBLIC HEALTH SCIENCE!

*You can't depend on your eyes when your imagination is out of focus*. Mark Twain

There are well over 25 million basic and clinical articles, books, and documents on cancer and vaccine topics. Despite the high cost of cancer sciences and therapeutics, using sophisticated, advanced, and specific technologies, the worthiness, caliber, and effectiveness of published studies, authored by those who occupy high positions and have accumulated scientific recognitions (eg, Nobel prizes), in “high impact” or “peer‐reviewed” journals are in decline. Too many expensive projects that are designed on reductionist approaches to cancer and vaccine sciences have failed the public. Numerous publications have been accepted or rejected because of political views of decision makers.^1^, ^2^, ^3^, ^4^, ^5^, ^6^, ^7^, ^8^, ^9^, ^10^, ^11^, ^12^, ^13^, ^14^, ^15^, ^16^, ^17^, ^18^, ^158^, ^167^, ^171^, ^223^ ‡‡‡‡‡‡‡‡‡‡’§§§§§§§§§§

Comparing the worthiness of publications in the past seven decades with those fundamental discoveries that stood the test of time, one can easily conclude that in the 18th or 19th century, the work of dedicated scientists who searched for the scientific truth to solve health‐biological problems were accomplished with limited resources and in the absence of highly modern technologies. As noted above, in the 20th century, it appears that the majority of pioneering studies are intellectually ignored or rejected for motives that diametrically oppose solving medical problems and improving public health and well‐being.

RETRACTED

The public is losing trust in conventional and “peer‐reviewed” publications that are supported and promoted by members of the establishment in governments, academia, and industries. Published data by independent and competent scientists are often downplayed, attacked, censored, or rejected by reviewers if the results do not fit the motives of the medical establishment. Professionals with financial ties to government and industry often label views of independent and competent professionals as a ‘threat’ to public health!^1^, ^2^, ^3^, ^4^, ^5^, ^6^, ^7^, ^8^, ^9^, ^10^, ^12^, ^13^, ^15^, ^16^, ^17^, ^22^, ^34^, ^71^, ^142^, ^145^, ^167^, ^196^, ^205^, ^206^, ^207^ (unpublished observations). Often independent, highly competent, and concerned professionals who are frustrated with the diseased condition of the money‐driven mentality of the medical system discuss or publish their views on different sites on Internet. In recent years, even quality independent scientific blogs are being controlled and censored under fabricated reasons (unpublished data).^8^, ^223^

## 10 FUTURE TRENDS OF MEDICAL SYSTEM FOR PUBLIC HEALTH: EXPANDING FACILITIES FOR CHRONIC DISEASE CARE AND PUSHING DRUGS OR VACCINES TO YOUNG AND OLD! CORPORATE PROFIT OVER PUBLIC HEALTH AND HUMANITY

*If people let government decide which food they eat and medicines they take, their bodies will soon be in as sorry a state as are the souls of those who live under tyranny*. Thomas Jefferson

Evidence for extension of establishment's power in forming a ‘global supreme leadership in medicine’ to minister and control public health comes from the recently intensified partnership between governments, Big Pharma, and venture capitalists“philanthropists.” On September 11, 2019, DHHS announced that it was sponsoring a health center [“*Awards More than $50 Million to Establish New Health Center Sites*”]. The announcement states that “*This new funding will increase access to health care for more than 400,000 new patients,…*”***********. At about the same time‐frame, to match taxpayers’ investment in ‘healthcare’ in expanding hospitals, vaccine manufacturers also announced hiring more staff for vaccine development†††††††††††. The Bill and Melinda Gates Foundation is also ‘investing’ millions in vaccinating children, in under‐developed countries and for corona virus vaccines globally‡‡‡‡‡‡‡‡‡‡‡!

RETRACTED

All of this sounds “great” except that vaccine injury courts have awarded billions of dollars to a small percentage of vaccine‐injured individuals who became aware of the relationship between vaccines and their illnesses or those who could legally afford to report their vaccine injuries. Available statistics on injury claims that are filed in the Federal Vaccine Injury Compensation Program (VICP) and other governmental and private organization programs show that public vaccinations with polio, smallpox, and Swine flu vaccines killed millions and left many more millions seriously injured, hospitalized, disabled and drug‐ dependent. At least 22 000 were killed after smallpox vaccination alone.^1^, ^2^, ^3^, ^4^, ^5^, ^6^, ^14^, ^17^ §§§§§§§§§§§ ^,^ ************ ^,^ †††††††††††† ^,^ *************

## 11 TWENTIETH CENTURY MEDICINE: SHIFTING DISEASE CATEGORIES TO INCREASE INDUCED DISEASES IN YOUNG AND OLD: WEALTH TRANSFER FROM the PUBLIC TO CORPORATE AMERICA!

*It's easier to fool people, than to convince them they have been fooled*. Mark Twain

A closer look at the current disease status of three to four generations in America, demonstrates that the major disease categories that are clinically, pathologically, and symptomatically identified as congenital, hereditary, neonatal and induced diseases have been shifted to increase the population toward induced diseases (Figures 1, 3–5).

Integration of the scattered data on epidemiological, environmental, clinical and basic research on developmental biology, inflammatory diseases, cancer and vaccine sciences, treatment options are outlined below^1^, ^2^, ^3^, ^4^, ^5^, ^6^, ^7^, ^8^, ^9^, ^10^, ^11^, ^12^, ^13^, ^14^, ^17^, ^24^, ^50^, ^71^, ^82^, ^86^, ^93^, ^119^, ^120^, ^128^, ^136^, ^150^, ^151^, ^152^, ^153^, ^155^, ^156^, ^176^, ^177^, ^182^, ^183^, ^184^, ^185^, ^203^, ^204^, ^205^, ^206^, ^207^, ^209^, ^210^, ^211^, ^212^, ^213^, ^214^, ^215^, ^216^, ^217^, ^218^, ^220^ ††††††††††††† ^,^ ‡‡‡‡‡‡‡‡‡‡‡‡‡ ^,^ §§§§§§§§§§§§§ ^,^ ************** ^:^

- Significant increase in the incidence of allergies, asthma, anaphylactic, anemia, emphysema, autoimmune and neuronal dysfunction, obesity, hypertension, diabetes and cardiovascular complications, stroke, gastritis, colitis, fibromyalgia, thyroiditis, lupus, Alzheimer's, Parkinson's, and site‐specific cancers in young and older adults. These disease incidences that require hospitalization and consumption of various drugs are at the level of near epidemic proportions. Asthma and allergies among children mandate that schools provide drugs, inhalers, and extremely expensive Epipens for asthmatic children;
- Increased incidence of autism spectrum disorder (ASD) is an example of a range of immune‐neuronal‐metabolic illnesses that sharply rose among young and growing population in the last few decades. In 1950s and 1960s, the estimated rates of reported autism were 1/10,000 in America. In 1990s this rate rose to 1/ 5000. In 2014, the CDC estimated that 1/45 children were autistic (NHIS data), a 30% increase from 1 of 150 in 2002 (just in 12 years!). In 2018, it was estimated that the rate of autism will be four times higher in boys compared with girls. Therefore, about one in five boys will suffer from ASD, not including the “unexplained” SIDS or other illnesses that are not reported as relevant. With the current trend, it is estimated that one in two boys (50%) could become autistic and manifest multiple physical and intellectual disabilities between 2025–2032.
- Increased population of individuals who suffer from neurodegenerative and autoimmune diseases and require long‐term consumption of drugs further complicate overall well being, productivity and hopefulness that youth will be able to contribute to the society;

RETRACTED

## 12 TOWARD UNIVERSAL AND SAFE VACCINE DEVELOPMENT: TIMELY CHALLENGES TO IMPROVE NATURAL IMMUNITY AND PUBLIC HEALTH

Intellectually, with the fundamental knowledge that effective immunity is responsible for defending and protecting the body against internal or external foreign (non‐self) elements (eg, infectious agents, pollutants, non‐functional proteins, mutated genes, defective or cancerous cells), it is hard to accept that medical decision makers could be so incompetent not to realize that research priorities should have been directed to a systematic understanding of the highly regulated multi‐layer complex bioelectrical signals that make up an effective immunity. By abusing fundamental information on the role of immunity, the medical system continues to conduct projects that chip away at immunity, even before completion of the immune system in the unborn or newborn or infant.

Pathogen‐specific vaccines and adjuvants seem to be “safer” new terms for drugging young and old populations and claiming that ‘vaccines promote immunity’!

Developing universal and safe vaccines that boost immunity and induce effective neutralizing antibodies and memory cells against a wide range of pathogenic structures [eg, envelope glycosylated proteins or glycoproteins (hemagglutinine‐rich structures), mannosyl‐rich proteins, glycolipids and related enzymes and receptor molecules] are yet to be seriously considered. Recent attempts toward ‘universal’ flu vaccines, while provide useful additional information and insights into shared or special structural and sub‐structural characteristics or compatibility among a few pathogens (eg, HIV, influenza) and the relation to host receptor glycoproteins and induction of immune responses (eg, IgGs) they are far from being considered as universal vaccines or safer treatment options^1^, ^32^, ^86^, ^96^, ^136^, ^210^, ^211^, ^212^ (manuscript in preparation). Such efforts for making a vaccine against pathogenic components of one infective family structure (eg, flu, SARS, or covid‐19) should not be claimed as ‘universal’. Outcomes of projects that are claimed as ‘universal’ vaccines are likely to present infinite response possibilities in vivo within the host site‐specific tissues. Depending on evolving pathogenic components (eg, molecular envelop glycoproteins, receptor or surface molecules) or host exposure tissue sites, as well as the health status or the age of individual in responding to pathogenic components, or how vaccines are developed (eg, composition of the incipient or engineered viral modifications [DNA or RNA]) could induce additional complicated and unknown electrochemical immune responses.^1^, ^5^, ^8^, ^12^, ^14^, ^19^, ^20^, ^22^, ^32^, ^62^, ^106^, ^129^, ^162^, ^172^, ^177^, ^185^, ^194^

## 13 DEFINITIONS OF HEALTH AND PHILANTHROPY IN TWENTIETH CENTURY: POWER TO PURCHASE PUBLIC HEALTH!

In 2011, Chris Hedges, a respected and independent journalist described the current health situation ‘*Industry's lobbyist and industry money wrote the healthcare bill*’††††††††††††††.

Unfortunately, the originalities of thinkers of the 18^th^ or 19^th^ century, who searched for the scientific truth suffered a great deal in the 20^th^ century. They were replaced by weakened ethical and moral standing and acceptance of egregious conflicts of interest tolerated and even encouraged by the medical might of the establishment, with its world's largest lobbying group who control healthcare, promote and mandate vaccines, and peddle drugs. Extensive debates, and controversies that were created by isolationists in cancer biology and treatment options as well as the emphasis on vaccines over immune system support resulted in conducting too many out‐of‐focus and expensive projects that repeatedly failed the public. Searching the truth in medical sciences, pioneers such as Pasteur, Rous, Metchnikoff, Ehrlich or Burnet employed highly intellectual logics by integrating and presenting credible discoveries of their era that stood the test of time. With limited resources and in the absence of modern technologies, these true scientists viewed infections as foundations of inflammatory chronic diseases. In the twentieth century, these logical, common sense and fundamental studies have been drastically altered, abused, and replaced by reductionist and chaotic tactics by profit‐power‐seeker mentalities of decision makers who disregard medical morality “to do no harm” in conducting medical sciences.^1^, ^2^, ^3^, ^4^, ^5^, ^6^, ^7^, ^8^, ^9^, ^10^, ^17^, ^18^

The medical system seems to have lost its soul to the power of blood (dark) money in the 20th century. Rockefeller Patent Medicine and Gates' Patent Vaccines altered definitions of health and philanthropy. Health definitions changed from the absence of disease to management of the disease by drugs/vaccines. Definitions of philanthropy have changed from doing good deeds to benefit society and humanity, to investing in diseases to benefit the investors. Disease investors and venture capitalists (‘philanthropists’) are giving more to their tax‐deductible foundations with the goal to collect a lot more! The overall outcomes of ‘philanthropists’ involvement in collaboration with Big Pharma and governments on public health projects, particularly cancer and vaccines may be summarized as:

- Shifted/increased in induced diseases in young and old;
- Reduced and disregarded medical morality, ethics and conflicts of interest in conducting projects;
- Prevented independent validation of research and clinical projects by competent professionals;
- Abused power to control a sick and drug‐dependent society for population growth control and the maintenance of a complacent work force;
- Transfer of wealth from the public to the disease investors (‘philanthropists’) and collaborators;

It is time to remind true ‘philanthropists’ to go back to do good deeds to benefit society. Supporting and improving hygiene, agriculture, clean drinking water, nutritional programs, and infrastructure in the third world or poor countries (eg, Samoa, Congo) where real human crisis/tragedies are happening would be considered doing good deed for humanity.

RETRACTED

Vaccine‐deficiency is not what the developed or undeveloped nations are suffering from! Immunologically, investing in vaccination (even if vaccines were ‘safe’) will not reduce diseases or death. Vaccines further complicate the disease status of poor people who suffer from malnutrition and lack of hygiene. The fear‐mongering tactics based on the threat of infectious diseases (eg, measles, Ebola, HPV, meningitis, flu, coronavirus) in developed or developing countries are an over‐exaggeration and cover‐up for pushing and selling drugs (vaccines) and controlling population growth. Malnutrition or bad nutrition (overeating of junk and unhealthy foods) are important factors in manifestations of diseases in developing‐poor nations or developed nations.^1^, ^3^, ^5^, ^7^, ^8^, ^172^, ^173^, ^174^ ‡‡‡‡‡‡‡‡‡‡‡‡‡‡’§§§§§§§§§§§§§§ Despite the fact that America invests the highest amount in advanced technologies and medical research and healthcare, the health status of Americans ranks last among other developed nations. The rates of reproduction and longevity are declining in America. Peculiarly, when the disease status in developed or under‐developed countries is compared, the overconsumption and overabundance of certain unhealthy foods, antibiotics, and drugs/vaccines, the overall health of Americans seems comparable with the levels of malnutrition and lack of hygiene in poor nations!

## 14 FUTURE DIRECTIONS: UNDERSTANDING AND PROMOTING ELECTROBIOLOGY OF EFFECTIVE IMMUNITY FOR MAINTENANCE OF HEALTH

The autonomic sympathetic and parasympathetic behaviors and circuitry that shape human immunity (adaptive, horizontal) cannot be explained by limited genomics (innate, perpendicular) that conventionally described certain inherited diseases (eg, sickle cell anemia, progeria).^221^, ^222^ Even these genomic diseases are potentially immune/inflammation‐based conditions that irreversibly affected parental/ancestral chromosomal/genetic structures and functions. Future studies should focus on a deep and systematic understanding of the complex electrobiology of immunity with time‐dependent and differential bioenergetics involving mitochondria and cytoplasm under a wide range of environmental and inflammatory conditions. Approaches to limit or control excessive activation of gene‐environment‐immunity are keys to assessing accurate risk formulations, preventing inducible diseases, developing universal safe vaccines, and promoting health, the most basic human right.^1^, ^5^, ^20^

RETRACTED

## 15 CONCLUDING REMARKS: HUMAN BODY IS NOT DRUG‐DEFICIENT, IT IS NOT VACCINE‐DEFICIENT!

*‘There could be no greater a heinous crime, than the premeditated withholding of truth from the masses, to the point of their injury or death*.(?)

In the last seven decades, the guardians of public health, instead of promoting health and preventing diseases, successfully managed to chip away the naturally synchronized and complex molecular dynamics of effective immunity and increased and shifted the population of induced diseases in young and old. Frequent use of drugs and pathogen‐specific vaccines are seeds of immune destruction that induce electrochemical sinkholes (mini electronic shocks) in time‐dependent circadian (biorhythms, the Yin‐Yang balance) of signal transduction mechanisms that primarily paralyze (exhaust) mitochondrial function, damage proton pumping and lead to initiation and progression of mild, moderate or severe diseases and death in young and old.

Heavy propaganda and demands to over‐vaccinate young and old populations, including the current fear‐mongering on the covid‐19 situation and lockdown (Medical Marshal Law) with the goal to vaccinate the public globally make us wonder whether “*Governments love pandemics… for the same reason they love war.…”* *************** or this lockdown is a political ideology that experiments how to strip public freedom and dignity “*replace freedom with the terrifying dreams of intellectuals*….”†††††††††††††††

Evidence was presented that (a) human body is not drug‐deficient or vaccine‐deficient; (b) current pathogen‐specific vaccines weaken immunity, not promote it; (c) current vaccines are new terms for drugging young and old; (d) safe, effective and universal vaccines that promote natural immunity and prevent diseases are yet to be seriously considered by the medical establishment.

Due to serious harms that continue to erode the public health, concerned independent scientific/medical experts, ethicists, attorneys, media, and policymakers are urged to take a closer look at intellectual crimes that the medical establishment has practiced against public health and to initiate appropriate actions before all hopes for a functional healthy society are lost. Policymakers, elected officials, and professionals should return to the common sense that our Forefathers valued and strive to serve the public for a ‘*more perfect Union’*.

Our universe can offer a lot more untapped resources to afford a larger human populations without the need to destroy and cause the extinction of human beings by inducing infertility and diseases to control population growth and shorten life span, as well as to continue to spawn a compliant and docile, drug‐dependent work force who can be eliminated at the push of syringe should they become expandable to their elite masters.

RETRACTED

It is a horrifying thought to choose between the less of the two evils for humanity; killing and destroying weaker nations by man‐made weapons under fabricated reasons for creating wars, or destroying public health and controlling the population by weaponizing cancer or over‐vaccinating the public under intellectual deceptions and claims of “war on cancer” or “vaccines are safe.” The real outcomes of either choice seem the same, transfer of wealth to warmongers, loss of precious lives and lack of respect and hope to save humanity.

These are challenging times for correcting the disease status that was created by Rockefeller medicine and continued by Gates vaccine. It requires a serious change of heart for policymakers and professionals, as well as a public awareness of the issues to help purge the deceptology in the cancer and vaccine sciences and hold the perpetrators of this deception responsible for fraudulent projects in the medical sciences.

After all ‘*Of one Essence is the human race, Thusly has Creation put the Base; One Limb impacted is sufficient, For all Others to feel the Mace’* Saadi Shirazi.

## CONFLICT OF INTEREST

No conflict of interest.

## Footnotes

* Governmental agencies that also indirectly participate in support of major decision making include DOD/DARPA, CIA, and Department of Agriculture. Examples of such collaboration include collaboration and support of CIA and DOD with NIH‐DHHS and medical schools to weaponize cancer for political purpose in 1940‐1950s [^8^]. Current collaboration between Homeland Security/Immigration and DHHS for detention of refugees at Mexican‐USA Border is another example of such collaboration.

† HPV and Meningitis with Offit, Caplan, et al Conference on “Achieving Childhood Vaccination Success in the U.S.: Expert Panel. May 16, 2016, https://www.youtube.com/watch?v = 07v0Yp05snA

‡ CHD, August 4, 2020 https://childrenshealthdefense.org/child-health-topics/known-culprit/vaccines-culprit/marylands-145-million-cervical-cancer-control-policy-fail/

§ The History of the Pharma Cartel, May 10, 2007 http://www.dr-rath-foundation.org/2007/05/the-history-of-the-pharma-cartel/

** Aseem Malhotra – 2019, .muckrack.com/aseem‐malhotra Why it's now time for a full public parliamentary inquiry into the controversial drug and fully expose the great cholesterol and statin con.

††
https://inews.co.uk/news/health/statins-review-nhs-government-chief-medical-adviser-norman-lamb/

§§ Josh Mazer, 2019 https://www.eyeonannapolis.net/2019/11/opinion-hpv-vaccine-incentive-payments-need-to-stop/

***
*Health Care System Compares Internationally*, The Commonwealth Fund, June 2014.

††† Luke Yamaguchi ‘The Dark Side of Vaccines’, 2020 https://www.darksidevaccines.com/how-to-end-vaccine-hesitancy/

‡‡‡ Maurice Hillman Interview (Aug 11, 2015): Vaccine pioneer admits adding cancer causing virus to Vaccine https://youtu.be/WeOt_uFPkg0

§§§ RFK Jr. Debate w Alan Dershowitz July 23,2020 https://www.facebook.com/PatrickBetDavid.Valuetainment/videos/213391659973360/

**** COVID‐19: No Law For Vaccine Compensation In India, Aug 3, 2020 https://www.mid-day.com/articles/covid19-no-law-for-vaccine-compensation-in-india/22914213

†††† Preventing a Covid‐19 pandemic‐Rapid response BMJ 2020;368:m810

‡‡‡‡ Arifa S Khan: FDA, 2/1/2018: Investigating viruses in cells used to make vaccines; and evaluating potential threat posed by transmission of viruses to humans https://www.fda.gov/vaccines-blood-biologics/biologics-research-projects/investigating-viruses-cells-used-make-vaccines-and-evaluating-potential-threat-posed-transmission. Accessed Aug 6, 2020.

§§§§ The Great Prostate Hoax ‐ SCIENCE TALK AND DISCUSSION 2017 https://youtu.be/lTjs0K-q5Is

***** In late 1980s, NEI/NIH abruptly discontinued support for extension of these pioneering studies and at the peak of author's productivity–Since 1998 at NCI/NIH, decision makers minimized, denied and downplayed author's submitted concepts and comprehensive proposals and her efforts to extend and promote the important role of inflammation/immunity in cancer research and therapy. See text.

††††† Obomsawin R: The Graphic Reality of Artificial Immunization, Natl Aboriginal Health Organization, Ottawa, Canada, November 2019.

‡‡‡‡‡ Deposition of Dr. Plotkin https://youtu.be/rGDNsqk0KR0?list = PLbDqqjs2g3N1F9FXps4JWJZzHDWI4mRjd –God Father of Vaccines under oat (1‐9 parts Deposition ‐2018).

§§§§§ Flu Season: U.S. Public Health Preparedness and Response. The US Congressional Subcommittee on Oversight and Investigations of the Committee on Energy and Commerce, Dec. 4, 2019. https://energycommerce.house.gov/committee-activity/hearings/hearing-on-flu-season-us-public-health-preparedness-and-response

******
http://mandateforchoice.com and https://www.ageofautism.com/2019/10/hpv-vaccine-for-all-the-obscene-public-farce-in-our-midst.html

††††††
https://healthit.ahrq.gov/sites/default/files/docs/publication/r18hs017045-lazarus-final-report-2011.pdf

‡‡‡‡‡‡ https://www.jeremyrhammond.com/2019/05/14/the‐cdcs‐criminal‐recommendation‐for‐a‐flu‐shot‐during‐pregnancy/

§§§§§§ The HighWire with Del Bigtree July 5, 2018 at 11:00 AM; James Neuenschwander, MD Interview– https://www.facebook.com/HighWireTalk/videos/404908657077423/

******* Robert F. Kennedy Jr. https://www.ageofautism.com/2020/11/the-problem-with-the-covid-vaccine-robert-f-kennedy-jr-explains-to-theo-von.html

††††††† Federal Food, Drug and Cosmetic (FD&C) Act‐Coronavirus Disease 2019 (COVID‐19) Emergency Use Authorizations for Medical Devices during Covid‐19, as of 11/3/2020

‡‡‡‡‡‡‡ Vaccines Licensed for Use in the United States | FDA www.fda.gov/vaccines-blood-biologics/vaccines/

§§§§§§§
https://pfe-pfizercom-d8-prod.s3.amazonaws.com/2020-09/C4591001_Clinical_Protocol.pdf

†††††††† Government Corruption AUGUST 20, 2020 Gardasil Lawsuit Claims HPV Vaccine Caused Teen Severe Injuries

‡‡‡‡‡‡‡‡ The Defender‐CHD November 19, 2020 Fourth Gardasil Lawsuit Against Merck Alleges Its HPV Vaccine Caused Debilitating Injuries

§§§§§§§§ Vaccine Components: https://www.cdc.gov/vaccines/vac-gen/additives.htm – or https://www.cdc.gov/vaccines/parents/ingredients.html

********* Common Ingredients in U.S. Licensed Vaccines https://www.fda.gov/vaccines-blood-biologics/safety-availability-biologics/commoningredients-us-licensed-vaccines: Accessed November 20, 2020

††††††††† Aluminum in Vaccines: What Everyone Needs to Know ‐ www.westonaprice.org/health-topics/vaccinations/

‡‡‡‡‡‡‡‡‡ Infant Immunity Part II: Aluminum, vaccines, and fetal brain development, with Dr. Suzanne Humphries www.youtube.com/watch?v=cdSCY7W-BUo and Infant Immunity with Suzanne Humphries and Hilary Butler; a four part series … 2015 www.youtube.com/playlist?list=PLgH2vCx5

§§§§§§§§§ Zostavax Shingles Lawsuits https://www.drugwatch.com/vaccines/zostavax/lawsuits/

********** Jon Heelevig (The Saker Blog) December 3, 2019. The Oligarch Takeover of US Pharma and Healthcare – And the Resulting Human Crisis http://thesaker.is/the-oligarch-takeover-of-us-pharma-and-healthcare-and-the-resulting-human-crisis/

‡‡‡‡‡‡‡‡‡‡ Tracker PD, Tennant J, Washington Post (August 1, 2019) https://www.washingtonpost.com/outlook/why‐we‐shouldnt‐take‐peer‐review‐as‐the‐gold‐standard/2019/08/01/fd90749a‐b229‐11e9‐8949‐5f36ff92706e_story.html?noredirect = on

§§§§§§§§§§ James Grundvig– Dr. Fauci and HCQ Exposed by the ‘Frontline Doctors’ https://vaxxter.com/dr-fauci-and-hcq-exposed-by-the-frontline-doctors/ 08/04/2020,

*********** U.S. Department of Health and Human Services ‘For Immediate Release September 11, 2019; DHHS Awards More than $50 Million to Establish New Health Center Sites ” HHS.Gov .

††††††††††† December 4, 2019 –WRALTechWire‐‘The drug giant announced a $57 million expansion of its vaccine manufacturing capability.’ https://www.wraltechwire.com/2019/12/04/merck-to-invest-57m-add-more-jobs-at-wilson-vaccine-plant/

‡‡‡‡‡‡‡‡‡‡‡ Bill & Melinda Gates Foundation www.gatesfoundation.org/Who‐We‐Are/General… and “Discover the Truth about Covid 19 ‐ Scientists are Warning Humanity!” https://www.stopworldcontrol.com/en/

§§§§§§§§§§§ https://www.jeremyrhammond.com/2019/10/17/how‐the‐media‐lie‐about‐why‐parents‐dont‐vaccinate/

************
https://pamw.pl/sites/default/files/inv_14_Gotzsche%20online.pdf

†††††††††††† HHS Awards Nearly $500 Million to Support Primary Health Care Workforce Nationwide (10/15/2020)

************* CDC/WHO will weaponize another 1918‐style Flu. In doing so, a vaccine will be created in miracle time to save (kill) humanity. https://www.brighteon.com/8879b5af-59b3-4ed3-98e6-f9037f22ade5

††††††††††††† Autism records https://www.cdc.gov/nchs/data/nhsr/nhsr087.pdf; https://www.cdc.gov/ncbddd/autism/data.html

‡‡‡‡‡‡‡‡‡‡‡‡‡ Auvin S, et al Altered vaccine‐induced immunity in children with Dravet syndrome. Epilepsia 2018, https://onlinelibrary.wiley.com/doi/full/10.1111/epi.14038

§§§§§§§§§§§§§ CDC Vaccine Information Sheet. 9/5/2006. https://www.cdc.gov/vaccines/pubs/vis/default.htm.

************** Erika Fry, 2019,Epidemic of Fear: How the Trouble‐Ridden Debut of a Breakthrough Vaccine Sparked a Panic’ fortune.com/longform/sanofi-dengue-fever-vaccine-dengvaxia

†††††††††††††† Chris Hedges on Death of the Liberal Class, 2011 https://youtu.be/NNrDej7aXMs

‡‡‡‡‡‡‡‡‡‡‡‡‡‡ Allie Buzett, Video, December 7, 2019, Dissolving Samoa Illusions, https://www.facebook.com/VaXismVideos/videos/2461661767410307/

§§§§§§§§§§§§§§ James Grundvig 12/10/2019 Measles Hysteria‐from Samoa to the Congo https://vaxxter.com/measles-vaccine-samoa-congo/

*************** Robert F Kennedy Jr, “Governments love pandemics. They love pandemics for the same reason they love war. Because it gives them the ability to impose control on the population that the population would otherwise NEVER accept…” Berlin, August 29, 2020.

††††††††††††††† Jeffrey A Tucker; Lockdown: The New Totalitarianism, Oct 1, 2020. https://www.aier.org/article/lockdown-the-new-totalitarianism/
